The article "A Learning Sparrow Search Algorithm" was published in 2021. Journal: Comput Intell Neurosci.

# A Learning Sparrow Search Algorithm

**DOI:** 10.1155/2021/3946958

**Published:** 2021-08-06

**Authors:** Chengtian Ouyang, Donglin Zhu, Fengqi Wang

**Affiliations:** School of Information Engineering, Jiangxi University of Science and Technology, Ganzhou, Jiangxi 341000, China

## Abstract

This paper solves the drawbacks of traditional intelligent optimization algorithms relying on 0 and has good results on CEC 2017 and benchmark functions, which effectively improve the problem of algorithms falling into local optimality. The sparrow search algorithm (SSA) has significant optimization performance, but still has the problem of large randomness and is easy to fall into the local optimum. For this reason, this paper proposes a learning sparrow search algorithm, which introduces the lens reverse learning strategy in the discoverer stage. The random reverse learning strategy increases the diversity of the population and makes the search method more flexible. In the follower stage, an improved sine and cosine guidance mechanism is introduced to make the search method of the discoverer more detailed. Finally, a differential-based local search is proposed. The strategy is used to update the optimal solution obtained each time to prevent the omission of high-quality solutions in the search process. LSSA is compared with CSSA, ISSA, SSA, BSO, GWO, and PSO in 12 benchmark functions to verify the feasibility of the algorithm. Furthermore, to further verify the effectiveness and practicability of the algorithm, LSSA is compared with MSSCS, CSsin, and FA-CL in CEC 2017 test function. The simulation results show that LSSA has good universality. Finally, the practicability of LSSA is verified by robot path planning, and LSSA has good stability and safety in path planning.

## 1. Introduction

In recent decades, the swarm intelligence optimization algorithm has been favored by many scholars due to its simple structure and high solving efficiency. Plenty of intelligent optimization algorithms have appeared continuously, such as monarch butterfly optimization (MBO) [1], smooth mount algorithm (SMA) [2], mother search algorithm (MSA) [3], hunter games search (HGS) [4], naked mole-rat algorithm (NMRA) [5], and Harris hawks optimization (HHO) [6]. Xue and Shen [7] proposed a sparrow search algorithm (SSA) that simulates the nature of sparrows foraging for food with the advantages of simple principle, fewer adjustment parameters, less programming difficulty, etc. Compared with grey wolf optimizer (GWO) [8], particle swarm optimization (PSO) [9], and genetic algorithm (GA) [10] in function optimization, it has better search results. Although excellent ability has been strongly confirmed, however, the SSA algorithm also has its own shortcomings. SSA is highly dependent on a certain role in the group and lacks learning ability. It is still easy to fall into the local optimum on high-dimensional complex problems.

At present, lots of scholars have carried out a series of studies so as to minify the shortcomings of the SSA itself. Scholars have studied and improved it separately, for the sake of further improving the optimization ability of the SSA. For example, Lu et al. [11] proposed a chaotic sparrow search algorithm (CSSA). The algorithm first used the tent mapping based on random variables to generate a better individual sparrow sequence and introduced tent perturbation as well as Gaussian mutation in the optimization process to carry out the solution found by the sparrow. The update prevents the algorithm from appearing premature; furthermore, the effectiveness of the algorithm is verified in the test function and image segmentation issues. At the same time, they stated an improved sparrow search algorithm (ISSA) to apply to the multithreshold image segmentation problem [12] and achieved meaningful results. In the process of algorithm optimization, the idea of a bird swarm algorithm is applied. The benchmark function and multithreshold image segmentation based on the variance between classes and Kapur entropy verify that the improved algorithm has strong search and development capabilities. Mao and Zhang [13] illustrated an improved sparrow search algorithm that combines Cauchy mutation and opposition-based learning. At first, a sin chaotic mechanism with an unlimited number of folds was used to initialize the population, and the previous generation global optimal solution was employed into the position update formula. For the aim of generating a new solution of higher quality, the information exchange of the algorithm was sped up, and the adaptive weight strategy was introduced to coordinate the local and global search capabilities, and the fusion Cauchy mutation and reverse learning strategy were utilized to perform disturbance mutation at the optimal position, which improved the ability of the algorithm to jump out of the local optimum. Eight test functions verify that the algorithm has been greatly improved in global optimization. Liu et al. [14], in order to better apply the SSA in 3D path planning, also adopted chaos strategies to enhance the diversity of the population and used adaptive inertial weights to balance the convergence speed and exploration capabilities of the algorithm. Finally, they adopted the Cauchy–Gaussian mutation strategy to get rid of the ability of the later algorithm stagnation, through the effect of planning the route, so that the improved SSA with a strong search ability is able to plan the route which is safer. Wang et al. [15] proposed a chaotic map sparrow search algorithm, which uses a dynamic adaptive weight mechanism to control the search range of the sparrow and finally uses reverse learning and Gaussian mutation to prevent the algorithm from falling into local optimality and balance the development of the algorithm and searchability as well. The 12 test functions proved that the improved algorithm has strong optimization capabilities. Zhang and Ding [16] also proposed a chaotic sparrow search algorithm, which strengthens the global search ability of the algorithm by introducing logistic mapping, adaptive hyperparameter, and mutation operation. The effectiveness of the algorithm is verified by the test function, and then, it is applied to the random configuration network. The results show that the proposed model has good regression accuracy.

The abovementioned authors have carried out a lot of experiments to verify the advantages of the proposed algorithm, but still there are some shortcomings:

1. Most papers put forward chaos theory. Chaos theory itself has uncertainty and cannot change the randomness of the algorithm. Therefore, a flexible search mechanism is needed to improve the situation.
2. The existing literature does not fundamentally change the optimization mechanism of the algorithm itself and lacks learning ability, so there is still a probability of falling into the local optimum when encountering high-dimensional complex problems.
3. At present, the improved algorithms are only tested on the function of the optimal value dimension 0, which lacks rationality and cannot fully explain the effectiveness of the algorithm.
4. Researchers only consider the update of the best location, but ignore the update of the worst location of SSA. The search method of SSA is closely related to the worst position.

Based on the above shortcomings, this paper proposes a learning sparrow search algorithm, with the help of lens reverse learning and random reverse learning to improve the learning ability of the algorithm and adapt to various complex models. The improved sine and cosine algorithm is used to guide the followers to update the position and improve the search precision. As a result, the local search based on the difference is used to update the optimal solution to improve the quality of the solution. LSSA is compared with CSSA, ISSA, SSA, beetle swarm optimization (BSO) [17], GWO, and PSO in 12 benchmark functions to verify the feasibility of the algorithm. In order to further verify its effectiveness and practicability, LSSA is compared with multistrategy serial cuckoo search algorithm (MSSCS) [18], CSsin [19], and firefly algorithm with courtship learning (FA-CL) [20] in CEC 2017 test function. All the three algorithms are verified in the CEC test function; finally, the results show that the LSSA algorithm has strong universality. The contributions of this paper are as follows:

- The fusion of two opposition-based learning strategies is proposed to improve the algorithm's global search capability
- An improved sine and cosine algorithm is proposed to improve the flexibility of the algorithm
- A local search based on the difference is proposed to improve the quality of the solution each time
- It has a good effect on the benchmark function and the CEC 2017 function and, at the same time, minifies the defect of the algorithm close to the origin
- LSSA is applied to robot path planning, and good results are achieved

This reminder of this paper is organized as follows.  Section 2 introduces the basic sparrow search algorithm and analyzes it.  Section 3 describes the process and validation of LSSA.  Section 4 shows the experiment and analysis of each algorithm on benchmark function and CEC 2017 test function. Section 5 provides discussion and future research directions.

## 2. Sparrow Search Algorithm

The SSA is divided into three phases: discoverer, follower, and investigator. As the name implies, the discoverer discovers food, searches for food, and provides direction for other individuals in the population. Therefore, the discoverer searches for a wide range of food, which accounts for 20% of the population. The location update formula for the discoverer is

(1) $$\begin{array}{c} X_{i,j}^{t+1}=\left\{\begin{array}{cc} X_{i,j}^{t}\cdot \;\exp\left(\frac{-h}{\alpha \cdot M}\right), & \text{if }R_{2}<\text{ST},\\ X_{i,j}^{t}+Q\cdot L, & \text{if }R_{2}\geq \text{ST}. \end{array}\right. \end{array}$$

In formula (1), *h* represents the current number of iterations, *M* is the maximum number of iterations, *X*_*i*,*j*_ denotes the current position of the *i*th sparrow in the *j*th dimension, *αε*[0,1] is a random number, *R*_2_ and ST represent warning and safety values, respectively, and when *R*_2_ < [0,1], ST < [0.5, 1], *Q* is a normal distribution of random numbers, and  *L* means 1 with all the elements of 1 × *D*. When *R*_2_ < ST, this indicates that the community environment is safe at this time, no predators are found around them, and the discoverer can perform a wide search mechanism. When *R*_2_ ≥ ST, this indicates that the individual within the group has discovered the predator and issued an alert, that all individuals in the group will make antipredatory actions, and that the discoverer will lead the follower to a safe location.

Followers perform food searches after the discoverer and neighborhood searches around the discoverer's location. Followers' location updates the formula as follows:

(2) $$\begin{array}{c} X_{i,j}^{t+1}=\left\{\begin{array}{cc} Q\cdot \;\exp\left(\frac{X_{\text{worst}}^{t}-X_{i,j}^{t}}{i^{2}}\right), & \text{if }i>\frac{n}{2},\\ X_{P}^{t+1}+\left|X_{i,j}^{t}-X_{P}^{t+1}\right|\cdot A^{+}\cdot L, & \text{otherwise}. \end{array}\right. \end{array}$$

In formula (2), *X*_*p*_ is the optimal position currently occupied by the discoverer, *X*_worst_ represents the worst position currently, and *A* is a matrix of 1 × *d*, where the value of each element is 1 or −1, and *A*^+^=*A*^*T*^(*AA*^*T*^)^−1^. When *i* > *n*/2, at this point, the sparrow population will counterattack when it senses danger.

Investigators are randomly selected individuals within the population. When predators invade, they will send out signals to make sparrows escape to a safe position. The behavior formula of investigators is as follows:

(3) $$\begin{array}{c} X_{i,j}^{t+1}=\left\{\begin{array}{cc} X_{\text{best}}^{t}+\beta \cdot \left|X_{i,j}^{t}-X_{\text{best}}^{t}\right|, & \text{if }f_{i}\neq f_{g},\\ X_{i,j}^{t}+K\cdot \left(\frac{\left|X_{i,j}^{t}-X_{\text{worst}}^{t}\right|}{\left(f_{i}-f_{w}\right)+\varepsilon }\right), & \text{if }f_{i}=f_{g}. \end{array}\right. \end{array}$$

In formula (3), *X*_best_ is the current global optimal location, *β* is the control step parameter, which is a random number with the normal distribution of mean value 0 and variance 1, *K* ∈ [− 1,1] is a random number, *f*_*i*_ is the fitness value of the sparrow, *f*_*g*_ and *f*_*w*_ are the best and worst fitness values in the current search range, respectively, and *ε* is the smallest real number to prevent the denominator from 0. When *f*_*i*_ ≠ *f*_*g*_, it means that the sparrow is at the boundary of the population and vulnerable to predators, so it needs to adjust its position. When *f*_*i*_=*f*_*g*_, this indicates that the sparrow individuals in the population are aware of the danger and need to be close to other sparrows in order to avoid the danger. *K* represents the direction of the sparrow movement and can also control the movement step.

### 2.1. Performance Analysis

SSA can be divided into three stages: discoverer, follower, and scout. From the three formulas, it can be seen that sparrow individuals depend on the search of the discoverer stage. The idea of adaptive weight is introduced in formula (1), but the adaptive weight still has defects in the face of high-dimensional complex functions and cannot open up a global vision. Therefore, it is necessary to make use of lens reverse learning and random reverse learning to dig out more hidden positions, but also increase the diversity of the population and make full preparation for the optimization in the later stage. Formula (2) has the defect of near-zero points; hence, nonlinear sine-cosine guidance is used to balance the local and global search. From the overall formula, the update distance between the front and back position of SSA is far, so the blind area between them becomes more. The local search based on the difference can improve the search precision and reduce the scope of the blind areas.

## 3. Learning Sparrow Search Algorithm

### 3.1. Opposition-Based Learning Strategy Based on Lens Principle

The discoverer leads other individuals to search for food, and the search method directly affects the overall search performance, so the discoverer must have a wide range and flexible search mechanism. To solve these problems, researchers have proposed the corresponding learning mechanism [21–23]. The general opposition-based learning strategy only solves the problem in a certain space [24–26], which still has monotonicity and risk of local optimization. As for this phenomenon, this paper provides two fusion opposition-based learning strategies to jointly improve the searchability of the discoverer. The opposition-based learning strategy based on the lens principle [27] is used to effectively update the location of the discoverer. The schematic diagram is shown in Figure 1. It is the opposition-based learning solution of the lens principle that is flexible and diverse, which is conducive to mining new solutions in the unknown area and increasing the diversity of the population. The principle is as follows:

In a certain space, suppose an individual *P* of height *h*, and individual *X*_*p*_ is the projection of individual *P* onto the *X*-axis. A lens of focal length *f* is placed on the base point position *O*, *O* is the midpoint of [*a*_*j*_, *b*_*j*_], and *a*_*j*_ and *b*_*j*_ represent the upper and lower limits of the *j*th dimension of the current solution. An image *P*′ of height *H*′ is obtained by the lens imaging process, and its projection on the coordinate axis is *X*_*P*_′ (reverse point). At this point, *X*_*P*_′ is the new individual generated by *X*_*p*_ through the opposition-based learning strategy based on the principle of lens imaging. The schematic diagram is shown in Figure 1.

As shown in Figure 1, the corresponding reverse point *X*_*P*_′ of individual *X*_*p*_ is obtained by taking *O* as the base point, which can be obtained by the lens imaging principle:

(4) $$\begin{array}{c} \frac{a+b/2-x_{p}}{x_{p}^{\prime }-a+b/2}=\frac{h}{h^{\prime }}. \end{array}$$

Let *h*/*h*′=*k*, and *k* is the scaling factor. After transformation, the reverse point can be obtained as

(5) $$\begin{array}{c} x_{p}^{\prime }=\frac{a+b}{2}+\frac{a+b}{2k}-\frac{x_{p}}{k}. \end{array}$$

Thus, when *k* = 1,

(6) $$\begin{array}{c} x_{p}^{\prime }=a+b-x_{p}. \end{array}$$

Formula (6) is called a general opposition-based learning strategy. From the above formulas, it is known that the general learning strategy is only a specific case of lens imaging opposition-based learning strategy, and the new individuals obtained by the general opposition-based learning strategy are fixed each time. In high-dimensional complex functions, new individuals with the fixed range also have the possibility of falling into the local optimum, and they are monotonic. By adjusting the parameter *K*, the new individuals based on the lens imaging learning strategy are dynamic, which improves the diversity of the population.

In this paper, we generalize the formula to the *d*-dimensional space:

(7) $$\begin{array}{c} x_{p}^{'j}=\frac{a_{j}+b_{j}}{2}+\frac{a_{j}+b_{j}}{2k}-\frac{x_{p}^{j}}{k}. \end{array}$$

In formula (7), *x*_*p*_^*j*^ and *x*_*p*_^′*j*^ are the *j*-dimensional components of *x*_*p*_ and *x*_*p*_′, respectively, and *a*_*j*_ and *b*_*j*_ represent the *j*-dimensional components of the upper and lower bounds of decision variables, respectively.

### 3.2. Opposition-Based Learning of the Worst Position

After the discoverer has searched, the worst position they get is not necessarily reliable. From formulas (2) and (3), it is known that the worst solution will affect the later stage of optimization, and the minimum value will give followers a better search range. This means that updating at the worst location is extremely important, which is also a point that scholars tend to ignore, only pursuing the optimal location and ignoring the integrity of the algorithm. This paper uses the random opposition-based mechanism to update the worst position; the specific formula is as follows:

(8) $$\begin{array}{c} x_{\text{worst}}^{\prime }\left(t\right)=a_{j}+\text{rand}\cdot \left(b_{j}-x_{\text{worst}}\right). \end{array}$$

### 3.3. Guidance Strategy Based on Improved Sine-Cosine Algorithm

In the follower location update formula of SSA, the follower searches the location of the follower immediately after the discoverer, and there are few dynamic parameters, so it is easy to limit the search range of sparrow population and blindness, which limits the searchability of the algorithm. To solve these problems, the strategy of sine-cosine guidance [28–30] is used in the follower stage to dynamically update the sparrow's individual position and expand the search scope by using the sine-cosine characteristics. The formula for updating follower positions with sine-cosine strategy is

(9) $$\begin{array}{c} X_{i}^{t+1}=\left\{\begin{array}{cc} X_{i}^{t}+r_{1}\cdot \;\sin\left(r_{2}\right)\cdot \left|r_{3}\cdot X_{P}^{t}-X_{i}^{t}\right|, & r_{4}\leq 0.5,\\ X_{i}^{t}+r_{1}\cdot \;\cos\left(r_{2}\right)\cdot \left|r_{3}\cdot X_{P}^{t}-X_{i}^{t}\right|, & r_{4}>0.5, \end{array}\right. \end{array}$$

(10) $$\begin{array}{c} r_{1}=a-t\cdot \frac{a}{M}. \end{array}$$

In the above formula, *r*_1_ is a parameter, determined by the number of iterations, and it is the key to determine the individual search range. As the number of iterations increases, *r*_1_ gets smaller and smaller, and the sparrow search range is also smaller and smaller. *a* is a constant, and the value of *a* in this paper is 2. *r*_2_ is a random number in the range [0, 2*π*], which determines the individual movement distance; *r*_3_ and *r*_4_ are random numbers in [0, 2] and [0, 1], respectively.

It can be seen from the formula that *r*_1_ uses linear decline to balance the search scope, but this approach is easily trapped into local optimal [31, 32] when facing high-dimensional complexity functions. Therefore, this paper adopts nonlinear decline to set *r*_1_ to balance local and global search [33]. The specific formula is as follows:

(11) $$\begin{array}{c} r_{1}=c+\frac{b}{\exp\left(4\times {\left(t/M\right)}^{4}\right)+1}. \end{array}$$

Among them, *b* is the fixed value of 0.1 and *c* is the regulating factor. After many experiments, when *c* = 0.9, the best effect is achieved. The introduction of an improved sine-cosine guidance strategy reduces the blindness of sparrow searches, accelerates information exchange between individuals in the population and those in the best and worst positions, and makes followers more purposeful in their searches. According to the characteristics of the above formulas, it is clear that the nonlinear decreasing parameters make the search more detailed and improve the convergence accuracy of the algorithm.

### 3.4. Local Search Based on Difference

Sparrows do not always get reliable optimal solutions for each search. Precocious phenomena occur when local extremes are encountered, which paralyzes the algorithm. In order to overcome this limitation, a differential local search is proposed to get rid of the attraction of local extremes and improve the quality of the solution. *P*_1_ and *P*_2_ are the historic optimal solution and the historic suboptimal solution of the population, respectively, in the process of SSA optimization. In this paper, the difference between the two solutions is used to guide *P*_1_ to search for a reliable optimal solution in the neighborhood. Differential guidance is accurate. This strategy enables sparrows to search between solutions to avoid missing high-quality solutions and blind searches. The implementation is as follows:

(12) $$\begin{array}{c} P_{1}^{\prime }=P_{1}+r\cdot C_{t}\cdot \left(P_{1}-P_{2}\right), \end{array}$$

where *P*_1_′ is the updated historical optimal solution, *r* is the uniform random number between [−1,1], and *C*_*t*_ is the local scaling factor. In the early stage of the algorithm, *P*_1_ is far away from the optimal solution, so a larger search range is needed to speed up the search speed. In the later stage, the distance is relatively short, and a smaller search range is needed to achieve higher mining accuracy. Therefore, the idea of inertia weight is introduced here, and the linear decline strategy is adopted. The range gradually shrinks as the number of iterations increases:

(13) $$\begin{array}{c} C_{t+1}=C_{t}\cdot \left(\frac{1-i}{M}\right). \end{array}$$

The greedy strategy is adopted to preserve the solution *P*_1_′ obtained by local search as follows:

(14) $$\begin{array}{c} P_{1}=\left\{\begin{array}{cc} P_{1}^{\prime }, & \text{fit}\left(P_{1}^{\prime }\right)>\text{fit}\left(P_{1}\right),\\ P_{1}, & \text{otherwise}, \end{array}\right. \end{array}$$

where fit(*x*) is the fitness value of *x*.

### 3.5. Learning Sparrow Search Algorithm

Compared with other algorithms, the SSA has better performance, but it has more random parameters, which leads to increased randomness and the probability of falling into the local extreme value. Therefore, a learning sparrow search algorithm is proposed in this paper. Two learning mechanisms are introduced in the finder stage, and the opposition-based learning based on the lens principle is adopted to enlarge the finder search range, improve the diversity of the population, and make the search method more flexible. In the follower stage, an improved sine and cosine strategy is introduced to adjust the sine and cosine by adopting a nonlinear decreasing method to reduce the blind search in the follower stage and make its search method more detailed. In the end, a local search based on difference is expounded to update the optimal solution and promote the quality of the solution during the iteration. The algorithm flow chart is shown in Figure 2. The specific pseudocode is shown in Algorithm 1.

### 3.6. Algorithm Validity Test

For making it obvious that LSSA improves the optimization mechanism of SSA and verify the scientificity and effectiveness of the LSSA algorithm, this paper takes the Schwefel function as an example and gives the individual distribution map of the two algorithms in the optimization process. Let the maximum number of iterations be 20 and the population number be 50. The function model diagram is shown in Figure 3. The individual distribution diagram of the two algorithms is shown in Figures 4 and 5.

From Figures 4 and 5, the LSSA algorithm converges fast, and most individuals are close to the optimal value, from the initial individual to the final individual distribution, while the SSA algorithm is still in a decentralized state, and the convergence speed is slow. Therefore, the LSSA algorithm's search mechanism is broad and detailed, and it can quickly find the best in the optimization process.

### 3.7. Time Complexity Analysis

Time complexity is an important index to judge an algorithm and determine the rationality of the algorithm. Let the population size of the algorithm in this paper be *P*, the maximum number of iterations be *M*, the dimension be *D*, and the ratio coefficients of discoverers and followers are *R*_1_ and *R*_2_, respectively. The time complexity of this paper is analyzed as follows:

From a macropoint of view, the time of the intelligent optimization algorithm is *O*(*P* × *M* × *D*), so is the sparrow search algorithm. The improved sparrow search algorithm not only does not change the structure of the algorithm but also increases the number of cycles; in this way, its time complexity is *O*(*P* × *M* × *D*), the same as the basic sparrow search algorithm.

From a microscopic point of view, the improved sparrow search algorithm increases a certain amount of computational complexity, and the opposition-based learning of the lens and the opposition-based learning of the worst position, respectively, increase the complexity of *O*(*R*_1_ × *P* × *M* × *D*) and *O*(*M*). The computational complexity of introducing the sine and cosine guiding mechanism is *O*(*R*_2_ × *P* × *M* × *D*), and the time complexity of introducing the local search based on the difference is *O*(*M*). It can be seen that the introduction of each strategy does not improve the order of magnitude of the sparrow search algorithm, and the time complexity is still *O*(*P* × *M* × *D*).

## 4. Benchmark Function Test

In order to better verify the optimization ability of the LSSA algorithm, this paper first selects 10 standard test functions for verification and compares them with the six algorithms of PSO, GWO, SSA, ISSA, CSSA, and BSO. BSO is a new and hot research fusion algorithm in recent years. The specific parameters are shown in the literature. The test function information table is shown in Table 1. *F*_1_–*F*_6_ are complex unimodal functions, and *F*_7_–*F*_9_ are high-dimensional complex functions; the rest is a fixed-dimensional function, where *F*_1_–*F*_9_ are tested in 30 and 100 dimensions. The population size and maximum iteration number of each algorithm are 100 and 500, respectively. The two learning factors in the particle swarm algorithm are *c*1 = *c*2 = 1.429 and weight *w* = 0.729, and each algorithm runs 30 times independently and calculates the best value (best), average (Ave), and standard deviation (std) of the running results. Three indicators comprehensively evaluate the optimization ability of each algorithm in function. For performance evaluation, simulations are performed on Windows 10 having Matlab 2019a, Intel(R) Core (TM) i5-10200H CPU @ 2.40 GHz with 16 GB RAM.

From Tables 2 and 3, the LSSA algorithm exhibits good optimization effects in both 30 and 100 dimensions. In the unimodal function, both LSSA and basic SSA algorithm can find the optimal value, indicating that the LSSA algorithm does not reduce the optimization ability of the algorithm itself, which shows the rationality of the LSSA algorithm. In the multimodal function, LSSA can show a strong optimization ability and has better convergence accuracy than other algorithms, and it does not significantly weaken the optimization ability of the LSSA algorithm in the 100 dimensions. In the fixed dimension function *F*_10_–*F*_12_, the LSSA algorithm has good stability and can find the same value almost every time, which is close to the theoretical optimal value.

In order to better describe the optimization process and convergence speed of each algorithm, the 30-dimensional convergence graph of each algorithm on each function is given, as shown in Figure 6.

As shown in Figure 6, LSSA has great advantages in the optimization speed and convergence accuracy of each function. It converges quickly on the unimodal function and has better antilocal attraction ability on the multimodal function. It can be seen that the LSSA algorithm gets rid of the constraints of the original algorithm's search mechanism and develops a better search space.

## 5. CEC 2017 Function Test

### 5.1. Algorithm Complexity

According to the requirements of CEC 2017 test standard, the complexity of the proposed algorithm needs to be calculated. Therefore, the following code is used to calculate the running time *T*_0_ of LSSA:

  for *i* = 1 : 1,000,000
 
*x* = 0.55 + double(*i*); *x* = *x* + *x*; *x* = *x*/2; *x* = *x* ∗ *x*; *x* = sqrt(*x*); *x* = log(*x*); *x* = exp(*x*); *x* = *x*/(*x* + 2);
  end

*T*_1_ is the calculation time of the F18 function under 200,000 evaluation times, and *T*_2_ is the average calculation time of the *F*_18_ function for 5 times under the same condition. The specific algorithm complexity is shown in Table 4.

### 5.2. Function Test

Experiments on benchmark functions alone cannot show the universality and effectiveness of the algorithm. To better illustrate the effectiveness of the LSSA algorithm and avoid the situation that the LSSA algorithm depends on the optimal value of 0, the algorithm is tested on CEC 2017 test function [34], and the number of evaluations is 10,000 ∗ dim, the dimension is 50 or 30, and the population number is 50. The test results of LSSA and SSA, CSSA, MSSCS, CSsin, and FA-CL are compared, and the specific parameters of each algorithm are shown in Table 5. Each algorithm runs 30 times independently and calculates five indexes of the results of each algorithm running on the function, namely, the best, the worst, the median, the mean, and the standard deviation. Each index can clearly reflect the optimization ability of each algorithm. The best value in each indicator is treated in bold font. At the same time, the Wilcoxon rank test is used to show whether there is a significant difference in each algorithm, and the experiment is carried out at the significance level of 5%. “ + ” means that the LSSA algorithm is better than other algorithms in the optimization effect, “−” means the opposite, and “ = ” means the same performance. Finally, the comparison of each algorithm is counted. The test results are shown in Tables 6 and 7.

From Tables 6 and 7, it is apparent that LSSA has a better optimization effect in both 30 and 50 dimensions, and each function is close to the theoretical optimal value, but the effect on the *F*_4_ function is poor. Although MSSCS and CSsin have better optimization effects, they show the very poor effects on *F*_1_, *F*_3_, and *F*_12-13_ in 50 dimensions. It can be seen that these two algorithms have limitations in this kind of problem. Other algorithms perform poorly and rarely approach the theoretical optimal value. From the statistical test, the LSSA algorithm is significantly different from other algorithms, showing better advantages, and some functions are similar to MSSCS and CSsin. Generally speaking, the LSSA algorithm has high universality and is more suitable for some complex optimization problems than other algorithms.

## 6. Robot Path Planning

This paper takes the classic robot path planning case to explore it. In path planning, each sparrow is a feasible path. Suppose that there are *n* feasible paths, and dimension *D* is determined by the number of lines from the starting point to the target point. The grid method is used for environment modeling, and the grid method is to use 1 × 1. According to the grid value, the obstacles in the equivalent position are calculated. Grid number 0 is defined as the feasible area, and 1 is the obstacle area. Then, the robot can plan the path on the grid assigned to 0, and dimension *D* is the column number of the grid map. The cost function of the path length of the *i*th sparrow is shown in the following equation:

(15) $$\begin{array}{c} f\left(x\right)=\overset{D-1}{\underset{j=1}{\sum }}\sqrt{{\left(x_{j+1}+x_{j}\right)}^{2}+{\left(y_{j+1}-y_{j}\right)}^{2}}. \end{array}$$

In equation (12), *j* is the *j*th dimension of a sparrow.

In order to better verify the practicability of the improved algorithm, LSSA is applied to robot path planning and SSA is used for comparative experiments. The number of populations is 50, and the number of iterations is 20. Other environmental parameters are consistent with the above CEC 2017 test. Each algorithm works in a 15 × 15 model, and the optimal route is shown in Figure 7. In order to eliminate the chance, each algorithm is tested 10 times, and the optimal route, average route, and worst route of each algorithm are counted. Three indicators are used to measure the stability and feasibility of each algorithm in this experiment. The optimization statistics of each algorithm are shown in Table 8.

It can be seen from Table 8 and Figure 7 that the minimum cost of LSSA planning is 19.7990, while the minimum cost of SSA is 25.4558. It can be seen that the route planning ability of LSSA is strong, and through the average value and the worst value, it can be seen that the route planned by LSSA has good stability. Therefore, LSSA has a good effect on robot path planning and can plan a more stable and safe route.

## 7. Conclusions

A learning sparrow search algorithm is proposed in this paper, overcoming the shortcomings of the SSA. The lens reverse learning and random reverse learning are introduced in the discoverer's position and the worst position, respectively, which make the discoverer's search method more flexible. Then, the improved sine-cosine guidance makes the follower search more detailed. Finally, the local search based on the difference is used to update the optimal solution, which improves the quality of each solution.

Through 12 standard test functions, LSSA is proved to be better than SSA, BSO, CSSA, ISSA, GWO, and PSO. At the same time, in order to avoid LSSA only depending on the zero point, this paper compares LSSA with MSSCS, CSsin, and FA-CL which have been verified by CEC function in recent years. The results show that the LSSA algorithm has good universality, while other algorithms have limitations in some functions. Finally, the practicability of LSSA is verified by robot path planning. The LSSA test effect is satisfying, but there are some shortcomings; for instance, during the function optimization process, the time consumption is large and cannot show the best effect on some functions of CEC 2017, showing an unstable effect. Of course, the increase of time is inevitable because we add workload. In the future, we need to do three aspects of work, the first is how to balance the time and optimization ability of the algorithm, the second is how to improve the stability of the algorithm on the basis of the previous, and the third is how to get a better application in practical complex engineering. On the contrary, we will also try to analyze and optimize in MBO, SMA, MSA, HGS, and HHO and better apply to practical problems.

## Figures and Tables

**Figure 1:** Lens schematic diagram.

**Figure 2:** Algorithm flowchart.

**Figure 3:** Schematic diagram of the Schwefel function.

**Figure 4:** Individual distribution of SSA. (a) SSA individual initialization map. (b) Individual distribution of SSA in 100 generations.

**Figure 5:** Individual distribution of LSSA. (a) LSSA individual initialization map. (b) Individual distribution of LSSA in 100 generations.

**Figure 6:** Convergence diagram of each algorithm. (a) *F*_1_. (b) *F*_2_. (c) *F*_3_. (d) *F*_4_. (e) *F*_5_. (f) *F*_6_. (g) *F*_7_. (h) *F*_8_. (i) *F*_9_. (j) *F*_10_. (k) *F*_11_. (l) *F*_12_.

**Figure 7:** Minimum path planning. (a) LSSA. (b) SSA.

**Algorithm 1:** The framework of the LSSA.

**Table 1:** Test function.

Function	Dimensions	Interval	Min
*F*_1_(*x*)=∑_*i*=1_^*n*^*x*_*i*_^2^	30/100	[−100, 100]	0
*F*_2_(*x*)=∑_*i*=1_^*n*^(∑_*j*=1_^*i*^*x*_*j*_)^2^	30/100	[−100, 100]	0
*F*_3_(*x*)=max_*i*_{|*x*_*i*_|, 1 ≤ *i* ≤ *n*}	30/100	[−100, 100]	0
*F*_4_(*x*)=∑_*i*=1_^*n*−1^[100(*x*_*i*+1_ − *x*_*i*_^2^)^2^+(*x*_*i*_ − 1)^2^]	30/100	[−30, 30]	0
*F*_5_(*x*)=∑_*i*=1_^*n*^([*x*_*i*_+0.5])^2^	30/100	[−100, 100]	0
*F*_6_(*x*)=∑_*i*=1_^*n*^*ix*_*i*_^4^+random[0，1)	30/100	[−1.28, 1.28]	0
$F_{7}\left(x\right)=\sum_{i=1}^{n}-x_{i}\sin\left(\sqrt{\left|x_{i}\right|}\right)$	30/100	[−500, 500]	−418.9829*n*
$F_{8}=\frac{\pi }{n}\left\{10\;\sin\left(\pi y_{1}\right)+\sum_{i=1}^{n-1}{\left(y_{i}-1\right)}^{2}\left[1+10\;\sin^{2}\left(\pi y_{i+1}\right)\right]+{\left(y_{n}-1\right)}^{2}\right\}+y_{i}=1+x_{i}+1/4$	30/100	[−50,50]	0
$u\left(x_{i},a,k,m\right)=\left\{\begin{array}{cc} k{\left(x_{i}-a\right)}^{m}, & x_{i}>a\\ 0, & -a<x_{i}<a\\ k{\left(-x_{i}-a\right)}^{m}, & x_{i}<-a \end{array}\right.$			
$F_{9}=418.9829n-\sum_{i=1}^{n}x_{i}\sin\left(\sqrt{\left|x_{i}\right|}\right)$	30/100	[−500, 500]	0
*F*_10_(*x*)=(1.5 − *x*_1_+*x*_1_*x*_2_)^2^+(2.25 − *x*_1_+*x*_1_*x*_2_^2^)^2^+(2.625 − *x*_1_+*x*_1_*x*_2_^3^)^2^	2	[−4.5, 4.5]	0
*F*_11_(*x*)=100(*x*_1_^2^ − *x*_2_)^2^+(*x*_1_ − 1)^2^+(*x*_3_ − 1)^2^+90(*x*_3_^2^ − *x*_4_)^2^+10.1((*x*_2_ − 1)^2^+(*x*_4_ − 1)^2^)+19.8(*x*_2_ − 1)(*x*_4_ − 1)	4	[−10,10]	0
$\begin{array}{c} F_{12}\left(x\right)={\left(0.002+\sum_{i=1}^{25}1/i+{\left(x_{1}-a_{1i}\right)}^{6}+{\left(x_{2}-a_{2i}\right)}^{6}\right)}^{-1}\text{ where}\\ a=\left(\begin{array}{cccccccccc} -32 & -16 & 0 & 16 & 32 & -32 & \ldots & 0 & 16 & 32\\ -32 & -32 & -32 & -32 & -32 & -16 & \ldots & 32 & 32 & 32 \end{array}\right) \end{array}$	2	[−65.536, 65.536]	0.998

**Table 2:** Comparison table of optimization effect of each algorithm (30 dimensions and fixed dimensions).

Function	Algorithm	Best	Ave	Std
*F*_1_(*x*)	LSSA	0	0	0
	BSO	1.8337	9.2351	8.0567
	CSSA	0	0	0
	ISSA	0	0	0
	SSA	0	0	0
	GWO	2.9726*E* − 42	9.9797*E* − 41	2.3113*E* − 40
	PSO	1.562*E* − 12	7.3034*E* − 11	1.5384*E* − 10

*F*_2_(*X*)	LSSA	0	0	0
	BSO	9.4317*E* − 10	5.8438	19.6417
	CSSA	0	0	0
	ISSA	0	0	0
	SSA	0	7.0603*E* − 92	3.8713*E* − 91
	GWO	1.2722*E* − 15	1.6521*E* − 11	5.6379*E* − 11
	PSO	2.4597	6.8764	4.6663

*F*_3_(*X*)	LSSA	0	0	0
	BSO	0.0417	1.5546	1.2080
	CSSA	0	0	0
	ISSA	0	3.7672*E* − 158	2.0634*E* − 157
	SSA	0	0	0
	GWO	1.0249*E* − 11	1.3528*E* − 10	1.3629*E* − 10
	PSO	0.06008	0.1756	0.08657

*F*_4_(*X*)	LSSA	1.3707*E* − 10	8.2877*E* − 06	1.5080*E* − 05
	BSO	233.8862	971.7400	841.0884
	CSSA	3.47*E* − 09	7.3760*E* − 05	1.0942*E* − 04
	ISSA	1.0562*E* − 07	1.2681*E* − 04	2.7208*E* − 04
	SSA	7.6415*E* − 09	3.1722*E* − 05	5.9606*E* − 05
	GWO	45.1861	46.6720	0.7848
	PSO	10.0094	102.2121	51.6541

*F*_5_(*X*)	LSSA	0	8.3405*E* − 32	1.7901*E* − 31
	BSO	0	3.6491*E* − 21	1.9700*E* − 20
	CSSA	2.4651*E* − 32	6.1469*E* − 29	1.7338*E* − 28
	ISSA	4.6878*E* − 29	1.3501*E* − 25	3.1929*E* − 25
	SSA	3.0814*E* − 32	2.7691*E* − 29	7.1572*E* − 29
	GWO	3.3762*E* − 07	1.0734*E* − 06	3.7183*E* − 07
	PSO	8.9363*E* − 32	1.9760*E* − 30	5.1909*E* − 30

*F*_6_(*X*)	LSSA	7.5495*E* − 06	3.6715*E* − 04	3.4039*E* − 04
	BSO	1.8821*E* − 03	8.0499*E* − 03	4.1052*E* − 03
	CSSA	1.5867*E* − 05	1.7275*E* − 04	1.2860*E* − 04
	ISSA	1.0528*E* − 05	2.2030*E* − 04	1.7169*E* − 04
	SSA	8.2819*E* − 06	1.6418*E* − 04	1.7567*E* − 04
	GWO	1.8171*E* − 04	5.6482*E* − 04	3.1679*E* − 04
	PSO	7.1929*E* − 03	1.8162*E* − 02	7.2361*E* − 03

*F*_7_(*X*)	LSSA	−12569.4866	−12151.0951	724.9186
	BSO	−12569.4866	−11205.6626	1020.4548
	ISSA	−10141.2347	−9080.1757	568.2124
	CSSA	−10022.9333	−9045.4556	574.4343
	SSA	−10258.1903	−8724.1633	718.2918
	GWO	−8262.1714	−6362.1144	709.0298
	PSO	−8324.1386	−6844.9716	752.6817

*F*_8_(*X*)	LSSA	3.5924*E* − 19	1.5863*E* − 15	3.8647*E* − 15
	BSO	0.1323	0.9448	0.6457
	CSSA	8.7326*E* − 15	2.3930*E* − 12	4.4060*E* − 12
	ISSA	1.9914*E* − 14	2.6662*E* − 12	5.2284*E* − 12
	SSA	3.4524*E* − 15	1.4887*E* − 11	3.5684*E* − 11
	GWO	1.4151*E* − 06	0.01468	9.2774*E* − 03
	PSO	6.4837*E* − 14	0.08643	0.2527

*F*_9_(*X*)	LSSA	4.9797*E* − 04	719.9689	812.9308
	BSO	3.8182*E* − 04	1272.5502	983.9231
	CSSA	−9082.3593	−8132.3934	763.6265
	ISSA	2191.2870	3460.1076	584.0178
	SSA	2587.7399	4017.9491	668.5352
	GWO	4518.4944	6050.6684	801.1268
	PSO	4601.8502	6257.0871	952.5740

*F*_10_(*X*)	LSSA	0	0	0
	BSO	0	0.3556	0.3866
	CSSA	0	1.8488*E* − 33	7.0361*E* − 33
	ISSA	0	0	0
	SSA	0	8.2173*E* − 33	4.5008*E* − 32
	GWO	3.2417*E* − 10	4.6721*E* − 08	3.9041*E* − 08
	PSO	0	0	0

*F*_11_(*X*)	LSSA	7.1484*E* − 17	1.0144*E* − 09	3.9939*E* − 09
	BSO	0	0.4704	1.7733
	CSSA	8.9576*E* − 13	1.1160*E* − 08	2.0300*E* − 08
	ISSA	2.8781*E* − 12	1.1195*E* − 07	2.9258*E* − 07
	SSA	2.6178*E* − 13	2.3804*E* − 07	1.0194*E* − 06
	GWO	3.5322*E* − 06	0.1966	0.4975
	PSO	6.6552*E* − 07	8.9930*E* − 04	8.7012*E* − 03

*F*_12_(*X*)	LSSA	0.998	0.998	0
	BSO	0.998	1.8886	1.4519
	CSSA	0.998	1.0641	0.3622
	ISSA	0.998	2.3662	3.3602
	SSA	0.998	2.4984	3.3421
	GWO	0.998	1.7255	0.9724
	PSO	0.998	1.1305	0.3436

**Table 3:** Comparison table of optimization effect of each algorithm (100 dimensions).

Function	Algorithm	Best	Ave	Std
*F*_1_(*x*)	LSSA	0	0	0
	BSO	195.6467	757.4745	391.4064
	CSSA	0	0	0
	ISSA	0	0	0
	SSA	0	0	0
	GWO	5.0820*E* − 18	2.6308*E* − 17	2.1089*E* − 17
	PSO	1.0668	12.4586	30.0289

*F*_2_(*X*)	LSSA	0	0	0
	BSO	0.0680	154.2623	315.1105
	CSSA	0	1.9637*E* − 206	0
	ISSA	0	0	0
	SSA	0	1.0517*E* − 212	0
	GWO	0.4399	11.8139	13.5850
	PSO	6831.9888	4185.5172	7632.0184

*F*_3_(*X*)	LSSA	0	0	0
	BSO	0.04267	1.7935	1.3896
	CSSA	0	1.1926*E* − 184	0
	ISSA	0	1.3563*E* − 144	7.4285*E* − 144
	SSA	0	1.9421*E* − 165	0
	GWO	2.0983*E* − 03	0.05209	0.0865
	PSO	7.3782	9.5753	1.2667

*F*_4_(*X*)	LSSA	2.9056*E* − 09	2.6894*E* − 05	2.4742*E* − 05
	BSO	1077.0368	1.3748*E* + 04	1.3239*E* + 04
	CSSA	4.2237*E* − 08	2.5499*E* − 04	3.4620*E* − 04
	ISSA	2.1761*E* − 07	2.6971*E* − 04	6.66094*E* − 04
	SSA	9.1735*E* − 09	7.9045*E* − 05	1.3805*E* − 04
	GWO	95.6787	96.9734	0.9208
	PSO	651.0884	3221.6846	6748.9024

*F*_5_(*X*)	LSSA	2.5013*E* − 11	9.1120*E* − 08	1.8203*E* − 07
	BSO	244.9986	777.9455	539.4453
	CSSA	4.0102*E* − 10	2.6523*E* − 07	3.6092*E* − 07
	ISSA	4.5456*E* − 11	1.9716*E* − 07	3.2439*E* − 07
	SSA	2.2699*E* − 10	9.0256*E* − 08	1.3690*E* − 07
	GWO	5.3138	6.7272	0.6593
	PSO	1.0675	4.4194	5.3378

*F*_6_(*X*)	LSSA	2.4150*E* − 06	1.2529*E* − 04	8.5801*E* − 05
	BSO	0.02903	0.1136	0.06599
	CSSA	3.137*E* − 05	3.1911*E* − 04	3.8926*E* − 04
	ISSA	1.1119*E* − 05	2.3439*E* − 04	1.9717*E* − 04
	SSA	2.4052*E* − 06	2.3133*E* − 04	1.8927*E* − 04
	GWO	9.4823*E* − 04	2.6521*E* − 03	1.1372*E* − 03
	PSO	0.4998	1.1219	0.3632

*F*_7_(*X*)	LSSA	−41082.3952	−36443.6428	4817.9562
	BSO	−40261.0069	−33461.9674	3925.7756
	ISSA	−26395.4326	−24633.4955	981.1676
	CSSA	−26934.0704	−24515.6636	1327.8950
	SSA	−27320.1874	−24637.4984	1078.1888
	GWO	−22404.2115	−16606.7711	2437.1531
	PSO	−23435.5935	−20056.7171	2277.0807

*F*_8_(*X*)	LSSA	1.1891*E* − 15	1.9561*E* − 12	3.1614*E* − 12
	BSO	0.1178	0.9327	0.6212
	CSSA	2.6323*E* − 15	1.1686*E* − 11	2.9995*E* − 11
	ISSA	2.4668*E* − 10	2.1636*E* − 07	1.1233*E* − 06
	SSA	2.1460*E* − 15	7.6085*E* − 12	2.1375*E* − 11
	GWO	2.1287*E* − 06	0.01593	9.1126*E* − 03
	PSO	2.3296*E* − 13	0.08298	0.1774

*F*_9_(*X*)	LSSA	0.4063	4843.1939	4063.8163
	BSO	1803.1299	7726.7640	4238.1062
	CSSA	1.4004*E* + 04	1.7119*E* + 04	1070.6257
	ISSA	2191.2870	3460.1076	584.0178
	SSA	1.4549*E* + 04	1.7425 + 04	1198.2007
	GWO	2.0063*E* + 04	2.4918*E* + 4	2683.4939
	PSO	1.6965*E* + 04	2.2306*E* + 04	4297.4782

**Table 4:** Complexity of the LSSA algorithm.

Dim	*T*_0_	*T*_1_	*T*_2_	|*T*_2_ − *T*_1_|/*T*_0_
30	0.0838	4.9412	3.9684	11.6085
50		9.1498	5.3006	54.1031

**Table 5:** Parameters of each algorithm.

Algorithm	SSA	CSSA	MSSCS	CSsin	FA-CL	LSSA
Parameter	Discoverers = 0.2 × *N* Investigators = 0.6 × *N*	Discoverers = 0.2 × *N* Investigators = 0.6 × *N*	*α* = 0.01 *β* = 1.5 *P*_*a*_ = 0.25 *C* = 0.2 PA_max_ = 0.35 PA_min_ = 0.25	*P*_max_ = 0.75 *P*_max_ = 0.25 Freq = 0.5	*α* = 0.01 *β*_min_ = 0.2 *β* = 1 *γ* = 1	Discoverers = 0.2 × *N* Investigators = 0.6 × *N*

**Table 6:** Test results of each algorithm in CEC 2017(dim = 30).

*F*	Index	SSA	CSSA	MSSCS	CSsin	FA-CL	LSSA
*F*_1_(*x*)	Best	**1.01E + 02**	1.03*E* + 02	1.00*E* + 10	1.00*E* + 10	8.21*E* + 05	1.10*E* + 02
	Worst	2.03*E* + 04	1.98*E* + 04	1.00*E* + 10	1.00*E* + 10	1.85*E* + 06	**1.86E + 04**
	Median	2.12*E* + 03	4.55*E* + 03	1.00*E* + 10	1.00*E* + 10	1.20*E* + 06	**1.84E + 03**
	Mean	4.80*E* + 03	6.27*E* + 03	1.00*E* + 10	1.00*E* + 10	1.28*E* + 06	**4.47E + 03**
	Std	5.74*E* + 03	5.94*E* + 03	0.00*E* + 00	0.00*E* + 00	2.96*E* + 05	**5.61E + 03**
	*P*	0.8073(=)	0.0484(+)	1.21*E* − 12(+)	1.21*E* − 12(+)	3.02*E* − 11(+)	

*F*_3_(*x*)	Best	3.52*E* + 02	**3.00E + 02**	3.08*E* + 02	3.14*E* + 02	8.98*E* + 02	**3.00E + 02**
	Worst	2.48*E* + 03	**3.00E + 02**	1.07*E* + 03	8.75*E* + 02	5.10*E* + 03	**3.00E + 02**
	Median	7.72*E* + 02	**3.00E + 02**	4.21*E* + 02	4.15*E* + 02	1.91*E* + 03	**3.00E + 02**
	Mean	9.05*E* + 02	**3.00E + 02**	4.82*E* + 02	4.55*E* + 02	2.25*E* + 03	**3.00E + 02**
	Std	2.93*E* + 01	1.77*E* − 03	1.64*E* + 01	1.27*E* + 02	2.17*E* + 01	**8.17 ***E* − **04**
	*P*	3.02*E* − 11(+)	0.0292(+)	3.02*E* − 11(+)	3.02*E* − 11(+)	3.02*E* − 11(+)	

*F*_4_(*X*)	Best	**4.00E + 02**	4.28*E* + 02	**4.00E + 02**	**4.00E + 02**	4.68*E* + 02	**4.00E + 02**
	Worst	5.21*E* + 02	5.17*E* + 02	4.89*E* + 02	4.67*E* + 02	5.32*E* + 02	**4.64E + 02**
	Median	4.74*E* + 02	4.90*E* + 02	4.84*E* + 02	4.04*E* + 02	5.15*E* + 02	**4.01E + 02**
	Mean	4.72*E* + 02	4.94*E* + 02	4.65*E* + 02	4.18*E* + 02	5.06*E* + 02	**4.09E + 02**
	Std	2.93*E* + 01	2.12*E* + 01	3.30*E* + 01	2.41*E* + 01	2.17*E* + 01	**1.64E + 01**
	*P*	1.41*E* − 09(+)	4.08*E* − 11(+)	1.10*E* − 08(+)	0.1241(=)	3.02*E* − 11(+)	

*F*_5_(*X*)	Best	5.69*E* + 02	6.14*E* + 02	5.36*E* + 02	**5.26E + 02**	6.36*E* + 02	5.54*E* + 02
	Worst	8.27*E* + 02	8.01*E* + 02	5.73*E* + 02	**5.69E + 02**	7.33*E* + 02	5.96*E* + 02
	Median	7.56*E* + 02	7.03*E* + 02	5.58*E* + 02	**5.53E + 02**	6.91*E* + 02	5.79*E* + 02
	Mean	7.53*E* + 02	7.01*E* + 02	5.57*E* + 02	**5.52E + 02**	6.84*E* + 02	5.77*E* + 02
	Std	5.71*E* + 01	4.74*E* + 01	**9.13E + 00**	9.40*E* + 00	2.59*E* + 01	1.08*E* + 01
	*P*	2.87*E* − 10(+)	3.02*E* − 11(+)	4.31*E* − 08(−)	1.17*E* − 09(−)	3.02*E* − 11(+)	

*F*_6_(*X*)	Best	6.13*E* + 02	6.09*E* + 02	**6.00E + 02**	**6.00E + 02**	6.28*E* + 02	**6.00E + 02**
	Worst	6.59*E* + 02	6.37*E* + 02	**6.00E + 02**	**6.00E + 02**	6.57*E* + 02	**6.00E + 02**
	Median	6.40*E* + 02	6.21*E* + 02	**6.00E + 02**	**6.00E + 02**	6.46*E* + 02	**6.00E + 02**
	Mean	6.40*E* + 02	6.21*E* + 02	**6.00E + 02**	**6.00E + 02**	6.45*E* + 02	**6.00E + 02**
	Std	1.12*E* + 02	6.40*E* + 00	1.08*E* + 01	6.79*E* − 03	9.34*E* + 01	**1.06E − 03**
	*P*	3.02*E* − 11(+)	3.02*E* − 11(+)	4.34*E* − 05(+)	0.002156(+)	3.02*E* − 11(+)	

*F*_7_(*X*)	Best	1.02*E* + 03	8.66*E* + 02	7.82*E* + 02	7.69*E* + 02	8.86*E* + 02	**7.60E + 02**
	Worst	1.37*E* + 03	1.26*E* + 03	8.27*E* + 02	8.07*E* + 02	1.26*E* + 03	**8.04E + 02**
	Median	1.27*E* + 03	9.66*E* + 02	8.07*E* + 02	7.92*E* + 02	1.07*E* + 03	**7.87E + 02**
	Mean	1.23*E* + 03	1.00*E* + 03	8.08*E* + 02	7.90*E* + 02	1.07*E* + 03	**7.86E + 02**
	Std	1.12*E* + 02	1.08*E* + 02	1.03*E* + 01	**8.80E + 00**	9.34*E* + 01	1.08*E* + 01
	*P*	3.02*E* − 11(+)	3.02*E* − 11(+)	8.48*E* − 09(+)	0.20620(=)	3.02*E* − 11(+)	

*F*_8_(*X*)	Best	9.22*E* + 02	8.64*E* + 02	8.42*E* + 02	8.40*E* + 02	8.74*E* + 02	**8.39E + 02**
	Worst	1.03*E* + 03	1.01*E* + 03	9.03*E* + 02	8.75*E* + 02	9.80*E* + 02	**8.77E + 02**
	Median	9.79*E* + 02	9.45*E* + 02	8.81*E* + 02	8.61*E* + 02	9.26*E* + 02	**8.60E + 02**
	Mean	9.75*E* + 02	9.42*E* + 02	8.78*E* + 02	8.59*E* + 02	9.23*E* + 02	**8.58E + 02**
	Std	2.41*E* + 01	2.93*E* + 01	1.51*E* + 01	1.00*E* + 01	2.42*E* + 01	**9.56E + 00**
	*P*	3.02*E* − 11(+)	7.39*E* − 11(+)	2.32*E* − 06(+)	0.6414(=)	3.34*E* − 11(+)	

*F*_9_(*X*)	Best	4.50*E* + 03	1.95*E* + 03	**9.00E + 02**	**9.00E + 02**	2.27*E* + 03	**9.00E + 02**
	Worst	5.47*E* + 03	5.86*E* + 03	9.49*E* + 02	**9.26E + 02**	6.12*E* + 03	9.93*E* + 02
	Median	5.39*E* + 03	5.15*E* + 03	9.05*E* + 02	9.05*E* + 02	4.53*E* + 03	**9.04E + 02**
	Mean	5.30*E* + 03	4.74*E* + 03	**9.07E + 02**	**9.07E + 02**	4.31*E* + 03	9.11*E* + 02
	Std	5.53*E* + 02	9.76*E* + 02	3.25*E* + 02	**7.14E + 00**	6.15*E* + 02	1.79*E* + 01
	*P*	3.02*E* − 11(+)	3.02*E* − 11(+)	0.66272(=)	0.9823(=)	3.02*E* − 11(+)	

*F*_10_(*X*)	Best	4.01*E* + 03	4.06*E* + 03	3.24*E* + 03	**2.31E + 03**	3.61*E* + 03	2.76*E* + 03
	Worst	6.07*E* + 03	5.93*E* + 03	4.81*E* + 03	3.95*E* + 03	6.19*E* + 03	**3.92E + 03**
	Median	5.07*E* + 03	4.71*E* + 03	4.10*E* + 03	3.38*E* + 03	5.19*E* + 03	**3.36E + 03**
	Mean	5.16*E* + 03	4.83*E* + 03	4.03*E* + 03	**3.35E + 03**	5.03*E* + 03	3.36*E* + 03
	Std	5.53*E* + 02	5.42*E* + 02	**3.25E + 02**	3.97*E* + 02	6.15*E* + 02	**3.25E + 02**
	*P*	3.02*E* − 11(+)	3.02*E* − 11(+)	1.01*E* − 08(+)	0.91170(=)	8.99*E* − 11(+)	

*F*_11_(*X*)	Best	1.18*E* + 03	1.14*E* + 03	**1.10E + 03**	1.11*E* + 03	1.16*E* + 03	1.11*E* + 03
	Worst	1.42*E* + 03	1.48*E* + 03	**1.14E + 03**	**1.14E + 03**	1.32*E* + 03	1.15*E* + 03
	Median	1.29*E* + 03	1.30*E* + 03	**1.12E + 03**	**1.12E + 03**	1.22*E* + 03	**1.12E + 03**
	Mean	1.30*E* + 03	1.30*E* + 03	**1.12E + 03**	**1.12E + 03**	1.23*E* + 03	**1.12E + 03**
	Std	6.50*E* + 01	7.29*E* + 01	8.27*E* + 00	7.78*E* + 00	4.49*E* + 01	**7.72E + 00**
	*P*	3.02*E* − 11(+)	3.34*E* − 11(+)	0.2707(=)	0.2588(=)	3.02*E* − 11(+)	

*F*_12_(*X*)	Best	4.55*E* + 04	1.32*E* + 04	1.75*E* + 04	**8.77E + 03**	1.29*E* + 06	2.07*E* + 04
	Worst	3.89*E* + 05	1.35*E* + 05	1.00*E* + 10	1.00*E* + 10	9.36*E* + 06	**1.05E + 05**
	Median	1.42*E* + 05	4.27*E* + 04	1.00*E* + 10	1.00*E* + 10	3.59*E* + 06	**5.48E + 04**
	Mean	1.64*E* + 05	4.83*E* + 04	5.67*E* + 09	**5.34E + 09**	4.18*E* + 06	**5.37E + 04**
	Std	**1.04E + 04**	2.58*E* + 04	6.46*E* + 09	5.07*E* + 09	3.20*E* + 04	2.18*E* + 04
	*P*	6.01*E* − 08(+)	1.83*E* − 05(+)	0.000386(+)	0.01727(+)	3.02*E* − 11(+)	

*F*_13_(*X*)	Best	1.45*E* + 03	2.79*E* + 03	1.67*E* + 03	**1.35E + 03**	5.41*E* + 04	**1.35E + 03**
	Worst	5.02*E* + 04	6.67*E* + 04	7.40*E* + 03	1.00*E* + 10	2.11*E* + 05	**1.57E + 03**
	Median	6.67*E* + 03	8.49*E* + 03	2.52*E* + 03	1.42*E* + 03	1.19*E* + 05	**1.41E + 03**
	Mean	1.05*E* + 04	1.44*E* + 04	2.89*E* + 03	6.67*E* + 08	1.13*E* + 05	**1.43E + 03**
	Std	1.04*E* + 04	1.84*E* + 04	1.18*E* + 03	2.54*E* + 09	3.20*E* + 04	**6.46E + 01**
	*P*	1.46*E* − 10(+)	3.02*E* − 11(+)	3.02*E* − 11(+)	0.1857(=)	3.02*E* − 11(+)	

*F*_14_(*X*)	Best	2.70*E* + 03	1.59*E* + 03	1.45*E* + 03	**1.43E + 03**	3.41*E* + 03	**1.43E + 03**
	Worst	4.36*E* + 04	1.74*E* + 04	1.49*E* + 03	**1.46E + 03**	5.26*E* + 04	**1.46E + 03**
	Median	9.44*E* + 03	4.69*E* + 03	1.47*E* + 03	**1.44E + 03**	2.86*E* + 04	**1.44E + 03**
	Mean	1.12*E* + 04	5.25*E* + 03	1.47*E* + 03	**1.44E + 03**	2.54*E* + 04	**1.44E + 03**
	Std	8.21*E* + 03	3.19*E* + 03	8.17*E* + 00	**8.03E + 00**	1.32*E* + 04	8.04*E* + 00
	*P*	3.02*E* − 11(+)	3.02*E* − 11(+)	6.70*E* − 11(+)	0.1580(=)	3.02*E* − 11(+)	

*F*_15_(*X*)	Best	2.01*E* + 03	1.79*E* + 03	1.57*E* + 03	**1.51E + 03**	1.94*E* + 04	**1.51E + 03**
	Worst	4.62*E* + 04	4.34*E* + 04	1.62*E* + 03	**1.53E + 03**	6.21*E* + 04	1.54*E* + 03
	Median	1.01*E* + 04	4.19*E* + 03	1.59*E* + 03	**1.52E + 03**	4.36*E* + 04	**1.52E + 03**
	Mean	1.62*E* + 04	9.43*E* + 03	1.59*E* + 03	**1.52E + 03**	4.08*E* + 04	**1.52E + 03**
	Std	3.42*E* + 02	1.06*E* + 04	1.26*E* + 01	**5.28E + 00**	3.21*E* + 02	2.08*E* + 02
	*P*	3.02*E* − 11(+)	3.02*E* − 11(+)	3.02*E* − 11(+)	0.1536(=)	3.02*E* − 11(+)	

*F*_16_(*X*)	Best	2.25*E* + 03	2.20*E* + 03	**1.71E + 03**	1.76*E* + 03	2.49*E* + 03	1.82*E* + 03
	Worst	3.62*E* + 03	3.39*E* + 03	2.45*E* + 03	**2.42E + 03**	3.68*E* + 03	**2.35E + 03**
	Median	2.96*E* + 03	2.77*E* + 03	**2.02E + 03**	2.05*E* + 03	3.07*E* + 03	2.03*E* + 03
	Mean	2.93*E* + 03	2.74*E* + 03	**2.05E + 03**	2.07*E* + 03	3.09*E* + 03	2.07*E* + 03
	Std	3.42*E* + 02	3.21*E* + 02	2.08*E* + 02	1.69*E* + 02	3.21*E* + 02	**1.53E + 02**
	*P*	6.70*E* − 11(+)	2.61*E* − 10(+)	0.5011(=)	0.6734(=)	3.02*E* − 11(+)	

*F*_17_(*X*)	Best	1.98*E* + 03	1.79*E* + 03	1.76*E* + 03	**1.73E + 03**	1.79*E* + 03	**1.73E + 03**
	Worst	2.88*E* + 03	2.71*E* + 03	**1.89E + 03**	1.99*E* + 03	2.54*E* + 03	**1.96E + 03**
	Median	2.47*E* + 03	2.23*E* + 03	1.79*E* + 03	1.80*E* + 03	2.08*E* + 03	**1.77E + 03**
	Mean	2.47*E* + 03	2.26*E* + 03	1.80*E* + 03	1.82*E* + 03	2.13*E* + 03	**1.79E + 03**
	Std	2.33*E* + 02	2.21*E* + 02	2.87*E* + 01	6.63*E* + 01	2.40*E* + 02	**5.62E + 01**
	*P*	3.02*E* − 11(+)	1.78*E* − 10(+)	0.005828(+)	0.07978(=)	9.76*E* − 10(+)	

*F*_18_(*X*)	Best	2.71*E* + 04	8.67*E* + 03	1.15*E* + 04	**1.87E + 03**	5.21*E* + 04	1.89*E* + 03
	Worst	5.02*E* + 05	2.96*E* + 05	7.70*E* + 04	2.81*E* + 03	6.73*E* + 05	**2.51E + 03**
	Median	1.15*E* + 05	1.07*E* + 05	3.44*E* + 04	**1.98E + 03**	2.36*E* + 05	**1.98E + 03**
	Mean	1.56*E* + 05	1.12*E* + 05	3.59*E* + 04	2.07*E* + 03	2.47*E* + 05	**2.01E + 03**
	Std	1.60*E* + 04	7.56*E* + 04	1.24*E* + 04	2.33*E* + 02	5.79*E* + 05	**2.63E + 00**
	*P*	3.02*E* − 11(+)	3.02*E* − 11(+)	3.02*E* − 11(+)	0.7844(=)	3.02*E* − 11(+)	

*F*_19_(*X*)	Best	2.06*E* + 03	2.27*E* + 03	1.94*E* + 03	**1.91E + 03**	2.16*E* + 05	**1.91E + 03**
	Worst	5.35*E* + 04	5.54*E* + 04	1.97*E* + 03	**1.92E + 03**	2.39*E* + 06	**1.92E + 03**
	Median	6.25*E* + 03	7.81*E* + 03	1.95*E* + 03	**1.91E + 03**	1.39*E* + 06	**1.91E + 03**
	Mean	1.37*E* + 04	1.49*E* + 04	1.95*E* + 03	**1.91E + 03**	1.32*E* + 06	**1.91E + 03**
	Std	1.60*E* + 04	1.56*E* + 04	7.42*E* + 00	**2.22E + 00**	5.79*E* + 05	2.63*E* + 00
	*P*	3.02*E* − 11(+)	3.02*E* − 11(+)	3.02*E* − 11(+)	0.7505(=)	3.02*E* − 11(+)	

*F*_20_(*X*)	Best	2.26*E* + 03	2.25*E* + 03	**2.02E + 03**	**2.02E + 03**	2.26*E* + 03	2.04*E* + 03
	Worst	3.05*E* + 03	2.82*E* + 03	2.34*E* + 03	**2.29E + 03**	2.69*E* + 03	2.31*E* + 03
	Median	2.58*E* + 03	2.40*E* + 03	2.16*E* + 03	2.15*E* + 03	2.31*E* + 03	**2.08E + 03**
	Mean	2.62*E* + 03	2.44*E* + 03	2.14*E* + 03	2.13*E* + 03	2.37*E* + 03	**2.12E + 03**
	Std	2.11*E* + 02	1.49*E* + 02	8.20*E* + 01	8.12*E* + 01	1.20*E* + 02	**6.43E + 01**
	*P*	4.50*E* − 11(+)	6.07*E* − 11(+)	5.01*E* − 01(=)	0.9351(=)	1.33*E* − 10(+)	

*F*_21_(*X*)	Best	2.42*E* + 03	2.39*E* + 03	**2.20E + 03**	**2.20E + 03**	2.37*E* + 03	**2.20E + 03**
	Worst	2.59*E* + 03	2.57*E* + 03	2.40*E* + 03	**2.38E + 03**	2.60*E* + 03	2.39**E + **03
	Median	2.50*E* + 03	2.47*E* + 03	2.38*E* + 03	2.36*E* + 03	2.45*E* + 03	**2.35E + 03**
	Mean	2.50*E* + 03	2.47*E* + 03	2.36*E* + 03	2.35*E* + 03	2.45*E* + 03	**2.34E + 03**
	Std	1.95*E* + 03	4.42*E* + 01	6.33*E* + 01	**4.11E + 01**	9.25*E* − 01	1.19*E* + 03
	*P*	3.02*E* − 11(+)	3.02*E* − 11(+)	2.13*E* − 05(+)	0.5691(=)	3.69*E* − 11(+)	

*F*_22_(*X*)	Best	**2.30E + 03**	**2.30E + 03**	**2.30E + 03**	**2.30E + 03**	2.31*E* + 03	**2.30E + 03**
	Worst	7.73*E* + 03	8.05*E* + 03	5.48*E* + 03	5.34*E* + 03	**2.31E + 03**	5.83*E* + 03
	Median	6.52*E* + 03	5.69*E* + 03	2.30*E* + 03	2.30*E* + 03	**2.31E + 03**	**2.30E + 03**
	Mean	5.96*E* + 03	4.81*E* + 03	3.00*E* + 03	3.10*E* + 03	**2.31E + 03**	2.53*E* + 03
	Std	1.95*E* + 03	2.19*E* + 03	1.19*E* + 03	1.19*E* + 03	**9.25 ***E* − **01**	8.77*E* + 02
	*P*	1.49*E* − 06(+)	3.91*E* − 02(+)	6.55*E* − 04(+)	8.89*E* − 02(+)	8.48*E* − 09(−)	

*F*_23_(*X*)	Best	2.77*E* + 03	2.71*E* + 03	2.66*E* + 03	2.67*E* + 03	2.82*E* + 03	**2.40E + 03**
	Worst	3.00*E* + 03	3.00*E* + 03	**2.73E + 03**	**2.73E + 03**	3.01*E* + 03	2.76*E* + 03
	Median	2.91*E* + 03	2.83*E* + 03	**2.71E + 03**	**2.71E + 03**	2.93*E* + 03	2.72*E* + 03
	Mean	2.90*E* + 03	2.84*E* + 03	2.71*E* + 03	2.71*E* + 03	2.92*E* + 03	**2.70E + 03**
	Std	5.30*E* + 01	6.12*E* + 01	**1.40E + 01**	1.49*E* + 01	5.79*E* + 01	6.38*E* + 01
	*P*	3.02*E* − 11(+)	1.96*E* − 10(+)	9.93*E* − 02(=)	1.22*E* − 01(=)	3.02*E* − 11(+)	

*F*_24_(*X*)	Best	2.95*E* + 03	2.92*E* + 03	2.86*E* + 03	2.86*E* + 03	2.94*E* + 03	**2.60E + 03**
	Worst	3.33*E* + 03	3.15*E* + 03	2.94*E* + 03	2.91*E* + 03	3.23*E* + 03	**2.91E + 03**
	Median	3.08*E* + 03	2.98*E* + 03	2.90*E* + 03	2.89*E* + 03	3.07*E* + 03	**2.88E + 03**
	Mean	3.10*E* + 03	3.00*E* + 03	2.90*E* + 03	2.89*E* + 03	3.07*E* + 03	**2.87E + 03**
	Std	1.52*E* + 01	5.59*E* + 01	**1.75E + 00**	1.30*E* + 01	2.19*E* + 01	7.35*E* + 01
	*P*	3.02*E* − 11(+)	3.02*E* − 11(+)	6.38*E* − 03(+)	9.63*E* − 02(=)	3.02*E* − 11(+)	

*F*_25_(*X*)	Best	**2.88E + 03**	**2.88E + 03**	**2.88E + 03**	**2.88E + 03**	2.89*E* + 03	**2.88E + 03**
	Worst	2.94*E* + 03	2.94*E* + 03	**2.89E + 03**	**2.89E + 03**	2.96*E* + 03	**2.89E + 03**
	Median	**2.89E + 03**	**2.89E + 03**	**2.89E + 03**	**2.89E + 03**	2.94*E* + 03	**2.89E + 03**
	Mean	2.90*E* + 03	**2.89E + 03**	**2.89E + 03**	**2.89E + 03**	2.93*E* + 03	**2.89E + 03**
	Std	1.52*E* + 01	1.32*E* + 01	1.75*E* + 00	1.61*E* + 00	2.19*E* + 01	**6.12E − 01**
	*P*	6.74*E* − 06(+)	6.38*E* − 03(+)	8.77*E* − 02(=)	8.77*E* − 01(=)	5.07*E* − 10(+)	

*F*_26_(*X*)	Best	3.67*E* + 03	2.90*E* + 03	**2.80E + 03**	**2.80E + 03**	2.83*E* + 03	**2.80E + 03**
	Worst	7.70*E* + 03	7.46*E* + 03	4.58*E* + 03	4.54*E* + 03	7.86*E* + 03	**4.28E + 03**
	Median	6.38*E* + 03	5.99*E* + 03	**2.90E + 03**	3.46*E* + 03	4.81*E* + 03	**2.90E + 03**
	Mean	6.33*E* + 03	5.64*E* + 03	3.33*E* + 03	3.60*E* + 03	4.77*E* + 03	**2.94E + 03**
	Std	8.67*E* + 02	1.37*E* + 03	6.98*E* + 02	7.26*E* + 02	1.87*E* + 03	**2.55E + 02**
	*P*	3.34*E* − 11(+)	3.32*E* − 06(+)	5.28*E* − 02(=)	6.19*E* − 01(=)	6.57*E* − 02(=)	

*F*_27_(*X*)	Best	3.22*E* + 03	3.20*E* + 03	3.18*E* + 03	**3.17E + 03**	3.36*E* + 03	**3.17E + 03**
	Worst	3.39*E* + 03	3.32*E* + 03	3.21*E* + 03	3.22*E* + 03	3.67*E* + 03	**3.21E + 03**
	Median	3.27*E* + 03	3.24*E* + 03	3.20*E* + 03	3.20*E* + 03	3.47*E* + 03	**3.20E + 03**
	Mean	3.27*E* + 03	3.25*E* + 03	3.20*E* + 03	3.20*E* + 03	3.48*E* + 03	**3.20E + 03**
	Std	4.95*E* + 01	2.64*E* + 01	3.67*E* + 01	1.08*E* + 01	9.39*E* + 00	**9.01E + 00**
	*P*	3.02*E* − 11(+)	1.21*E* − 10(+)	9.05*E* − 02(=)	5.94*E* − 02(=)	3.02*E* − 11(+)	

*F*_28_(*X*)	Best	**3.10E + 03**	**3.10E + 03**	**3.10E + 03**	**3.10E + 03**	3.18*E* + 03	**3.10E + 03**
	Worst	3.25*E* + 03	3.26*E* + 03	3.21*E* + 03	**3.20E + 03**	3.21*E* + 03	3.26*E* + 03
	Median	3.11*E* + 03	**3.10E + 03**	**3.10E + 03**	**3.10E + 03**	3.20*E* + 03	**3.10E + 03**
	Mean	3.14*E* + 03	3.14*E* + 03	3.11*E* + 03	**3.12E + 03**	3.20*E* + 03	3.14*E* + 03
	Std	4.95*E* + 01	6.30*E* + 01	3.67*E* + 01	3.92*E* + 01	**9.39E + 00**	5.94*E* + 01
	*P*	1.33*E* − 02(+)	8.07*E* − 01(=)	5.27*E* − 06(−)	6.29*E* − 05(−)	1.00*E* − 03(+)	

*F*_29_(*X*)	Best	3.80*E* + 03	3.60*E* + 03	3.32*E* + 03	3.29*E* + 03	3.88*E* + 03	**3.28E + 03**
	Worst	4.69*E* + 03	4.43*E* + 03	3.63*E* + 03	**3.56E + 03**	4.84*E* + 03	3.63*E* + 03
	Median	4.09*E* + 03	3.98*E* + 03	3.47*E* + 03	3.44*E* + 03	4.34*E* + 03	**3.41E + 03**
	Mean	4.16*E* + 03	4.00*E* + 03	3.46*E* + 03	3.44*E* + 03	4.33*E* + 03	**3.43E + 03**
	Std	2.40*E* + 02	2.05*E* + 02	8.23*E* + 01	**7.44E + 01**	2.72*E* + 02	7.74*E* + 01
	*P*	3.02*E* − 11(+)	3.69*E* − 11(+)	1.05*E* − 01(=)	5.49*E* − 01(=)	3.02*E* − 11(+)	

*F*_30_(*X*)	Best	5.80*E* + 03	5.30*E* + 03	7.68*E* + 03	**5.27E + 03**	1.15*E* + 06	5.33*E* + 03
	Worst	2.42*E* + 04	2.13*E* + 04	1.17*E* + 04	**6.27E + 03**	4.46*E* + 06	6.93*E* + 03
	Median	9.94*E* + 03	7.31*E* + 03	9.56*E* + 03	5.74*E* + 03	2.21*E* + 06	**5.67E + 03**
	Mean	1.10*E* + 04	9.26*E* + 03	9.70*E* + 03	**5.74E + 03**	2.52*E* + 06	5.80*E* + 03
	Std	4.95*E* + 01	4.15*E* + 03	1.08*E* + 03	2.81*E* + 02	8.37*E* + 05	**3.67E + 01**
	*P*	2.37*E* − 10(+)	2.88*E* − 06(+)	3.02*E* − 11(+)	0.9117(=)	3.02*E* − 11(+)	
+/ = /−		28/1/0	28/1/0	18/9/2	5/22/2	27/1/1	

**Table 7:** Test results of each algorithm in CEC 2017(dim = 50).

*F*	Index	SSA	CSSA	MSSCS	CSsin	FA-CL	LSSA
*F*_1_(*x*)	Best	1.06*E* + 02	1.02*E* + 02	1.00*E* + 10	1.00*E* + 10	3.48*E* + 06	**1.01E + 02**
	Worst	2.08*E* + 04	2.29*E* + 04	1.00*E* + 10	1.00*E* + 10	6.99*E* + 06	**9.93E + 03**
	Median	2.31*E* + 03	1.15*E* + 03	1.00*E* + 10	1.00*E* + 10	5.22*E* + 06	**1.19E + 03**
	Mean	3.05*E* + 03	2.98*E* + 03	1.00*E* + 10	1.00*E* + 10	5.16*E* + 06	**2.39E + 03**
	Std	4.04*E* + 03	4.48*E* + 03	**0.00E + 00**	**0.00E + 00**	7.96*E* + 05	2.74*E* + 03
	*P*	0.3870(=)	0.7171(=)	1.21*E* − 12(+)	1.21*E* − 12(+)	3.02*E* − 11(+)	

*F*_3_(*x*)	Best	1.18*E* + 03	3.01*E* + 02	1.47*E* + 04	1.25*E* + 04	2.25*E* + 04	**3.00E + 02**
	Worst	1.02*E* + 04	3.09*E* + 02	4.03*E* + 04	3.89*E* + 04	7.91*E* + 04	**3.01E + 02**
	Median	5.66*E* + 03	3.03*E* + 02	2.51*E* + 04	1.99*E* + 04	4.52*E* + 04	**3.00E + 02**
	Mean	5.60*E* + 03	3.03*E* + 02	2.63*E* + 04	2.22*E* + 04	4.48*E* + 04	**3.00E + 02**
	Std	2.82*E* + 03	1.55*E* + 00	6.32*E* + 03	7.45*E* + 03	4.63*E* + 01	**1.09E − 01**
	*P*	3.02*E* − 11(+)	3.02*E* − 11(+)	3.02*E* − 11(+)	3.02*E* − 11(+)	3.02*E* − 11(+)	

*F*_4_(*X*)	Best	4.01*E* + 02	4.08*E* + 02	**4.00E + 02**	4.09*E* + 02	4.75*E* + 02	**4.00E + 02**
	Worst	6.17*E* + 02	7.30*E* + 02	6.61*E* + 02	**5.39E + 02**	6.86*E* + 02	5.40*E* + 02
	Median	4.72*E* + 02	5.33*E* + 02	5.46*E* + 02	**4.29E + 02**	6.03*E* + 02	4.73*E* + 02
	Mean	4.88*E* + 02	5.35*E* + 02	5.27*E* + 02	**4.47E + 02**	5.87*E* + 02	4.60*E* + 02
	Std	6.85*E* + 01	6.81*E* + 01	7.76*E* + 01	3.46*E* + 01	4.63*E* + 01	**3.38E + 01**
	*P*	2.52*E* − 01(=)	3.16*E* − 05(+)	1.77*E* − 03(+)	3.15*E* − 02(−)	9.92*E* − 11(+)	

*F*_5_(*X*)	Best	8.19*E* + 02	8.19*E* + 02	6.21*E* + 02	5.84*E* + 02	7.43*E* + 02	**5.75E + 02**
	Worst	9.22*E* + 02	9.11*E* + 02	6.89*E* + 02	**6.74E + 02**	9.00*E* + 02	6.90*E* + 02
	Median	8.77*E* + 02	8.64*E* + 02	6.55*E* + 02	6.36*E* + 02	7.94*E* + 02	**6.34E + 02**
	Mean	8.69*E* + 02	8.66*E* + 02	6.54*E* + 02	**6.34E + 02**	7.97*E* + 02	6.35*E* + 02
	Std	2.72*E* + 01	2.24*E* + 01	1.94*E* + 01	2.25*E* + 01	3.72*E* + 01	**1.99E + 01**
	*P*	3.02*E* − 11(+)	3.02*E* − 11(+)	1.06*E* − 03(+)	9.23*E* − 01(=)	3.02*E* − 11(+)	

*F*_6_(*X*)	Best	6.38*E* + 02	6.33*E* + 02	**6.00E + 02**	**6.00E + 02**	6.43*E* + 02	**6.00E + 02**
	Worst	6.65*E* + 02	6.63*E* + 02	**6.00E + 02**	**6.00E + 02**	6.67*E* + 02	**6.00E + 02**
	Median	6.53*E* + 02	6.50*E* + 02	**6.00E + 02**	**6.00E + 02**	6.60*E* + 02	**6.00E + 02**
	Mean	6.53*E* + 02	6.49*E* + 02	**6.00E + 02**	**6.00E + 02**	6.59*E* + 02	**6.00E + 02**
	Std	7.26*E* + 00	9.15*E* + 00	2.81*E* − 02	**9.62E − 03**	1.36*E* + 02	2.70*E* − 02
	*P*	3.02*E* − 11(+)	3.02*E* − 11(+)	3.03*E* − 02(+)	2.39*E* − 04(−)	3.02*E* − 11(+)	

*F*_7_(*X*)	Best	1.30*E* + 03	1.17*E* + 03	8.65*E* + 02	**8.35E + 02**	1.27*E* + 03	8.59*E* + 02
	Worst	1.82*E* + 03	1.82*E* + 03	9.60*E* + 02	9.36*E* + 02	1.99*E* + 03	**9.26E + 02**
	Median	1.75*E* + 03	1.56*E* + 03	9.14*E* + 02	9.02*E* + 02	1.70*E* + 03	**8.95E + 02**
	Mean	1.68*E* + 03	1.52*E* + 03	9.16*E* + 02	8.98*E* + 02	1.67*E* + 03	**8.96E + 02**
	Std	1.37*E* + 02	1.94*E* + 02	2.30*E* + 01	2.08*E* + 01	1.36*E* + 02	**1.44E + 01**
	*P*	3.02*E* − 11(+)	3.02*E* − 11(+)	1.58*E* − 04(+)	3.63*E* − 01(=)	3.02*E* − 11(+)	

*F*_8_(*X*)	Best	1.10*E* + 03	1.08*E* + 03	8.83*E* + 02	**8.79E + 02**	1.03*E* + 03	9.20*E* + 02
	Worst	1.25*E* + 03	1.26*E* + 03	9.76*E* + 02	**9.65E + 02**	1.20*E* + 03	1.00*E* + 03
	Median	1.19*E* + 03	1.19*E* + 03	9.30*E* + 02	**9.29E + 02**	1.10*E* + 03	9.63*E* + 02
	Mean	1.18*E* + 03	1.19*E* + 03	9.32*E* + 02	**9.30E + 02**	1.10*E* + 03	9.61*E* + 02
	Std	4.05*E* + 01	4.04*E* + 01	1.80*E* + 01	2.23*E* + 01	3.66*E* + 01	**1.79E + 01**
	*P*	3.02*E* − 11(+)	3.02*E* − 11(+)	4.11*E* − 07(−)	1.61*E* − 06(−)	3.02*E* − 11(+)	

*F*_9_(*X*)	Best	1.08*E* + 04	1.03*E* + 04	9.38*E* + 02	9.22*E* + 02	1.07*E* + 04	**9.01E + 02**
	Worst	1.46*E* + 04	1.38*E* + 04	1.77*E* + 03	**1.18E + 03**	2.04*E* + 04	1.66*E* + 03
	Median	1.31*E* + 04	1.30*E* + 04	1.12*E* + 03	**1.01E + 03**	1.52*E* + 04	1.06*E* + 03
	Mean	1.29*E* + 04	1.27*E* + 04	1.16*E* + 03	**1.03E + 03**	1.54*E* + 04	1.10*E* + 03
	Std	8.52*E* + 02	8.73*E* + 02	1.86*E* + 02	**6.47E + 01**	8.38*E* + 02	1.83*E* + 02
	*P*	3.02*E* − 11(+)	3.02*E* − 11(+)	1.45*E* − 01(=)	3.18*E* − 01(=)	3.02*E* − 11(+)	

*F*_10_(*X*)	Best	6.33*E* + 03	6.32*E* + 03	5.62*E* + 03	4.96*E* + 03	6.23*E* + 03	**4.67E + 03**
	Worst	9.53*E* + 03	1.00*E* + 04	7.60*E* + 03	**6.57E + 03**	9.50*E* + 03	6.86*E* + 03
	Median	8.14*E* + 03	7.73*E* + 03	6.47*E* + 03	5.81*E* + 03	8.16*E* + 03	**5.70E + 03**
	Mean	8.12*E* + 03	7.82*E* + 03	6.52*E* + 03	5.77*E* + 03	8.02*E* + 03	**5.75E + 03**
	Std	6.74*E* + 02	8.10*E* + 02	4.72*E* + 02	**4.02E + 02**	8.38*E* + 02	6.04*E* + 02
	*P*	1.07*E* − 09(+)	3.08*E* − 08(+)	5.46*E* − 06(+)	2.57*E* − 07(+)	3.35*E* − 08(+)	

*F*_11_(*X*)	Best	1.20*E* + 03	1.21*E* + 03	**1.14E + 03**	1.18*E* + 03	1.25*E* + 03	**1.14E + 03**
	Worst	1.58*E* + 03	1.41*E* + 03	1.18*E* + 03	1.40*E* + 03	1.42*E* + 03	**1.17E + 03**
	Median	1.36*E* + 03	1.29*E* + 03	1.16*E* + 03	1.29*E* + 03	1.33*E* + 03	**1.15E + 03**
	Mean	1.37*E* + 03	1.30*E* + 03	1.16*E* + 03	1.30*E* + 03	1.34*E* + 03	**1.15E + 03**
	Std	8.19*E* + 01	4.72*E* + 01	9.46*E* + 00	5.71*E* + 01	3.85*E* + 01	**8.10E + 00**
	*P*	3.02*E* − 11(+)	3.02*E* − 11(+)	3.34*E* − 03(+)	8.19*E* − 01(=)	3.02*E* − 11(+)	

*F*_12_(*X*)	Best	4.63*E* + 05	**1.22E + 05**	1.00*E* + 10	1.00*E* + 10	1.04*E* + 07	1.68*E* + 05
	Worst	3.71*E* + 06	3.83*E* + 06	1.00*E* + 10	1.00*E* + 10	5.74*E* + 07	**2.25E + 06**
	Median	1.30*E* + 06	9.68*E* + 05	1.00*E* + 10	1.00*E* + 10	2.55*E* + 07	**9.61E + 05**
	Mean	1.64*E* + 06	1.35*E* + 06	1.00*E* + 10	1.00*E* + 10	2.57*E* + 07	**1.09E + 06**
	Std	9.69*E* + 05	9.69*E* + 05	**0.00E + 00**	**0.00E + 00**	1.06*E* + 05	5.84*E* + 05
	*P*	4.68*E* − 02(+)	4.64*E* − 01(=)	1.21*E* − 12(+)	1.21*E* − 12(+)	3.02*E* − 11(+)	

*F*_13_(*X*)	Best	4.81*E* + 03	**3.09E + 03**	1.00*E* + 10	1.00*E* + 10	2.31*E* + 05	4.40*E* + 03
	Worst	5.11*E* + 04	**4.77E + 04**	1.00*E* + 10	1.00*E* + 10	6.39*E* + 05	4.81*E* + 04
	Median	1.90*E* + 04	1.15*E* + 04	1.00*E* + 10	1.00*E* + 10	4.16*E* + 05	**1.03E + 04**
	Mean	2.35*E* + 04	1.66*E* + 04	1.00*E* + 10	1.00*E* + 10	4.02*E* + 05	**1.55E + 04**
	Std	1.54*E* + 04	1.36*E* + 04	0.00*E* + 00	0.00*E* + 00	1.06*E* + 05	**1.16E + 04**
	*P*	4.84*E* − 02(+)	9.82*E* − 01(=)	1.21*E* − 12(+)	1.21*E* − 12(+)	3.02*E* − 11(+)	

*F*_14_(*X*)	Best	2.89*E* + 03	4.47*E* + 03	1.64*E* + 03	1.50*E* + 03	2.95*E* + 04	**1.46E + 03**
	Worst	2.11*E* + 05	1.68*E* + 05	1.93*E* + 03	1.59*E* + 03	4.22*E* + 05	**1.55E + 03**
	Median	2.70*E* + 04	4.00*E* + 04	1.78*E* + 03	1.54*E* + 03	1.14*E* + 05	**1.50E + 03**
	Mean	4.95*E* + 04	4.51*E* + 04	1.77*E* + 03	1.54*E* + 03	1.35*E* + 05	**1.50E + 03**
	Std	4.91*E* + 04	4.08*E* + 04	6.03*E* + 01	**1.73E + 01**	8.34*E* + 04	2.07*E* + 01
	*P*	3.02*E* − 11(+)	3.02*E* − 11(+)	3.02*E* − 11(+)	4.69*E* − 08(+)	3.02*E* − 11(+)	

*F*_15_(*X*)	Best	2.05*E* + 03	2.48*E* + 03	1.77*E* + 03	1.61*E* + 03	7.52*E* + 04	**1.56E + 03**
	Worst	3.68*E* + 04	3.60*E* + 04	3.15*E* + 03	**2.00E + 03**	2.26*E* + 05	3.01*E* + 03
	Median	1.48*E* + 04	1.89*E* + 04	1.92*E* + 03	**1.68E + 03**	1.48*E* + 05	1.69*E* + 03
	Mean	1.65*E* + 04	1.66*E* + 04	1.99*E* + 03	**1.72E + 03**	1.50*E* + 05	1.77*E* + 03
	Std	1.05*E* + 04	9.16*E* + 03	2.56*E* + 02	**1.03E + 02**	4.96*E* + 02	2.66*E* + 02
	*P*	3.69*E* − 11(+)	4.08*E* − 11(+)	9.53*E* − 07(+)	8.19*E* − 01(=)	3.02*E* − 11(+)	

*F*_16_(*X*)	Best	2.94*E* + 03	2.87*E* + 03	**2.08E + 03**	2.14*E* + 03	3.04*E* + 03	2.30*E* + 03
	Worst	4.63*E* + 03	4.17*E* + 03	3.21*E* + 03	3.35*E* + 03	4.71*E* + 03	**3.18E + 03**
	Median	3.68*E* + 03	3.53*E* + 03	2.70*E* + 03	**2.62E + 03**	4.12*E* + 03	2.79*E* + 03
	Mean	3.77*E* + 03	3.59*E* + 03	2.67*E* + 03	**2.62E + 03**	3.96*E* + 03	2.78*E* + 03
	Std	4.72*E* + 02	3.67*E* + 02	2.93*E* + 02	3.02*E* + 02	4.96*E* + 02	**2.24E + 02**
	*P*	1.78*E* − 10(+)	2.37*E* − 10(+)	1.91*E* − 01(=)	1.56*E* − 02(−)	5.49*E* − 11(+)	

*F*_17_(*X*)	Best	2.35*E* + 03	2.72*E* + 03	2.11*E* + 03	**2.01E + 03**	3.00*E* + 03	**2.01E + 03**
	Worst	4.02*E* + 03	4.18*E* + 03	2.71*E* + 03	**2.70E + 03**	4.31*E* + 03	2.78*E* + 03
	Median	3.42*E* + 03	3.43*E* + 03	2.47*E* + 03	**2.31E + 03**	3.57*E* + 03	2.43*E* + 03
	Mean	3.37*E* + 03	3.39*E* + 03	2.43*E* + 03	**2.32E + 03**	3.56*E* + 03	2.40*E* + 03
	Std	4.05*E* + 02	3.57*E* + 02	1.74*E* + 02	**1.62E + 02**	3.02*E* + 02	1.92*E* + 02
	*P*	2.87*E* − 10(+)	4.08*E* − 11(+)	6.10*E* − 01(=)	7.01*E* − 02(=)	3.02*E* − 11(+)	

*F*_18_(*X*)	Best	9.41*E* + 04	7.26*E* + 04	**2.51E + 04**	6.30*E* + 04	3.20*E* + 05	4.45*E* + 04
	Worst	9.83*E* + 05	4.50*E* + 05	3.71*E* + 05	**2.02E + 05**	2.59*E* + 06	2.64*E* + 05
	Median	2.48*E* + 05	1.63*E* + 05	1.17*E* + 05	1.16*E* + 05	1.23*E* + 06	**8.99E + 04**
	Mean	2.78*E* + 05	1.75*E* + 05	1.39*E* + 05	1.27*E* + 05	1.23*E* + 06	**1.01E + 05**
	Std	1.61*E* + 05	8.15*E* + 04	8.07*E* + 04	**3.92E + 04**	1.18*E* + 06	4.43*E* + 04
	*P*	8.89*E* − 10(+)	1.75*E* − 05(+)	3.92*E* − 02(+)	3.85*E* − 03(+)	3.02*E* − 11(+)	

*F*_19_(*X*)	Best	2.98*E* + 03	2.38*E* + 03	2.06*E* + 03	1.96*E* + 03	1.03*E* + 05	**1.93E + 03**
	Worst	4.46*E* + 04	4.43*E* + 04	2.73*E* + 03	2.03*E* + 03	3.66*E* + 06	**2.00E + 03**
	Median	2.05*E* + 04	1.69*E* + 04	2.29*E* + 03	1.99*E* + 03	1.39*E* + 06	**1.95E + 03**
	Mean	2.28*E* + 04	2.13*E* + 04	2.32*E* + 03	1.99*E* + 03	1.61*E* + 06	**1.95E + 03**
	Std	1.63*E* + 04	1.32*E* + 04	1.37*E* + 02	**1.57E + 01**	1.18*E* + 06	1.60*E* + 01
	*P*	3.02*E* − 11(+)	3.02*E* − 11(+)	3.02*E* − 11(+)	3.20*E* − 09(+)	3.02*E* − 11(+)	

*F*_20_(*X*)	Best	2.72*E* + 03	2.61*E* + 03	2.25*E* + 03	2.30*E* + 03	2.50*E* + 03	**2.15E + 03**
	Worst	3.87*E* + 03	3.80*E* + 03	2.84*E* + 03	2.86*E* + 03	3.82*E* + 03	**2.72E + 03**
	Median	3.23*E* + 03	3.19*E* + 03	2.62*E* + 03	2.56*E* + 03	3.20*E* + 03	**2.44E + 03**
	Mean	3.28*E* + 03	3.20*E* + 03	2.60*E* + 03	2.56*E* + 03	3.21*E* + 03	**2.46E + 03**
	Std	3.19*E* + 02	3.65*E* + 02	**1.38E + 02**	1.39*E* + 02	3.14*E* + 02	1.50*E* + 02
	*P*	3.34*E* − 11(+)	1.33*E* − 10(+)	6.20*E* − 04(+)	9.07*E* − 03(+)	1.21*E* − 10(+)	

*F*_21_(*X*)	Best	2.50*E* + 03	2.55*E* + 03	2.41*E* + 03	**2.40E + 03**	2.44*E* + 03	2.41*E* + 03
	Worst	2.85*E* + 03	2.86*E* + 03	2.50*E* + 03	2.47*E* + 03	2.78*E* + 03	**2.46E + 03**
	Median	2.68*E* + 03	2.68*E* + 03	2.47*E* + 03	**2.43E + 03**	2.63*E* + 03	**2.43E + 03**
	Mean	2.69*E* + 03	2.68*E* + 03	2.46*E* + 03	**2.43E + 03**	2.61*E* + 03	**2.43E + 03**
	Std	9.83*E* + 01	7.97*E* + 01	2.11*E* + 01	1.87*E* + 01	2.24*E* + 03	**1.44E + 01**
	*P*	3.02*E* − 11(+)	3.02*E* − 11(+)	1.47*E* − 07(+)	8.30*E* − 01(=)	6.07*E* − 11(+)	

*F*_22_(*X*)	Best	8.06*E* + 03	8.10*E* + 03	**2.30E + 03**	**2.30 ***E* + **03**	2.32*E* + 03	**2.30E + 03**
	Worst	1.21*E* + 04	1.11*E* + 04	8.54*E* + 03	**8.35E + 03**	1.20*E* + 04	9.50*E* + 03
	Median	9.61*E* + 03	9.92*E* + 03	**7.47E + 03**	7.55*E* + 03	1.03*E* + 04	8.38*E* + 03
	Mean	9.79*E* + 03	9.66*E* + 03	6.95*E* + 03	**6.90E + 03**	9.82*E* + 03	7.88*E* + 03
	Std	1.08*E* + 03	8.33*E* + 02	1.65*E* + 03	1.91*E* + 03	2.24*E* + 03	**1.60E + 03**
	*P*	3.96*E* − 08(+)	1.10*E* − 08(+)	2.28*E* − 05(−)	4.08*E* − 05(−)	3.96*E* − 08(+)	

*F*_23_(*X*)	Best	3.02*E* + 03	3.09*E* + 03	2.82*E* + 03	**2.73E + 03**	3.06*E* + 03	2.74*E* + 03
	Worst	3.48*E* + 03	3.44*E* + 03	2.94*E* + 03	**2.91E + 03**	3.59*E* + 03	2.94*E* + 03
	Median	3.18*E* + 03	3.27*E* + 03	2.87*E* + 03	**2.87E + 03**	3.31*E* + 03	2.89*E* + 03
	Mean	3.22*E* + 03	3.26*E* + 03	**2.87E + 03**	**2.87E + 03**	3.31*E* + 03	2.89*E* + 03
	Std	1.18*E* + 02	7.68*E* + 01	**2.76E + 01**	3.47*E* + 01	1.28*E* + 02	3.69*E* + 01
	*P*	3.02*E* − 11(+)	3.02*E* − 11(+)	2.16*E* − 03(−)	2.38*E* − 03(−)	3.02*E* − 11(+)	

*F*_24_(*X*)	Best	3.22*E* + 03	3.17*E* + 03	**2.99E + 03**	3.00*E* + 03	3.32*E* + 03	3.00*E* + 03
	Worst	3.71*E* + 03	3.58*E* + 03	3.15*E* + 03	**3.14E + 03**	3.78*E* + 03	**3.14E + 03**
	Median	3.36*E* + 03	3.40*E* + 03	3.07*E* + 03	3.06*E* + 03	3.54*E* + 03	**3.05E + 03**
	Mean	3.38*E* + 03	3.39*E* + 03	3.08*E* + 03	3.06*E* + 03	3.53*E* + 03	**3.05E + 03**
	Std	1.19*E* + 02	9.85*E* + 01	**3.43E + 01**	3.68*E* + 01	3.30*E* + 01	3.59*E* + 01
	*P*	3.02*E* − 11(+)	3.02*E* − 11(+)	5.57*E* − 03(+)	5.30*E* − 01(=)	3.02*E* − 11(+)	

*F*_25_(*X*)	Best	**2.96E + 03**	2.98*E* + 03	**2.96E + 03**	**2.96E + 03**	3.01*E* + 03	**2.96E + 03**
	Worst	3.11*E* + 03	3.12*E* + 03	3.08*E* + 03	3.06*E* + 03	3.14*E* + 03	**3.03E + 03**
	Median	3.07*E* + 03	3.08*E* + 03	3.03*E* + 03	2.98*E* + 03	3.12*E* + 03	**3.02E + 03**
	Mean	3.05*E* + 03	3.07*E* + 03	3.03*E* + 03	2.99*E* + 03	3.11*E* + 03	**3.00E + 03**
	Std	3.83*E* + 01	2.94*E* + 01	3.74*E* + 01	2.99*E* + 01	3.30*E* + 01	**2.53E + 01**
	*P*	7.60*E* − 07(+)	2.87*E* − 10(+)	1.32*E* − 04(+)	8.19*E* − 01(=)	1.29*E* − 09(+)	

*F*_26_(*X*)	Best	**2.90E + 03**	**2.90E + 03**	**2.90E + 03**	**2.90E + 03**	1.03*E* + 04	**2.90E + 03**
	Worst	1.13*E* + 04	1.13*E* + 04	5.58*E* + 03	**5.52E + 03**	1.40*E* + 04	5.80*E* + 03
	Median	**2.90E + 03**	6.53*E* + 03	5.13*E* + 03	4.87*E* + 03	1.19*E* + 04	**2.90E + 03**
	Mean	5.81*E* + 03	6.49*E* + 03	5.02*E* + 03	4.18*E* + 03	1.19*E* + 04	**3.95E + 03**
	Std	3.69*E* + 03	3.61*E* + 03	**6.09E + 02**	1.15*E* + 03	9.27*E* + 02	1.24*E* + 03
	*P*	1.86*E* − 01(=)	8.07*E* − 01(=)	2.61*E* − 02(+)	2.12*E* − 01(=)	3.02*E* − 11(+)	

*F*_27_(*X*)	Best	3.35*E* + 03	3.43*E* + 03	3.24*E* + 03	3.20*E* + 03	3.80*E* + 03	**3.17E + 03**
	Worst	4.07*E* + 03	3.84*E* + 03	3.38*E* + 03	3.34*E* + 03	5.08*E* + 03	**3.33E + 03**
	Median	3.57*E* + 03	3.57*E* + 03	3.30*E* + 03	3.27*E* + 03	4.44*E* + 03	**3.26E + 03**
	Mean	3.57*E* + 03	3.62*E* + 03	3.31*E* + 03	**3.26E + 03**	4.47*E* + 03	**3.26E + 03**
	Std	1.45*E* + 02	1.16*E* + 02	4.11*E* + 01	**3.49E + 01**	4.30*E* + 01	3.81*E* + 01
	*P*	3.02*E* − 11(+)	3.02*E* − 11(+)	3.18*E* − 04(+)	8.88*E* − 01(=)	3.02*E* − 11(+)	

*F*_28_(*X*)	Best	**3.26E + 03**	**3.26E + 03**	**3.26E + 03**	**3.26E + 03**	3.29*E* + 03	**3.26E + 03**
	Worst	3.32*E* + 03	3.43*E* + 03	3.31*E* + 03	**3.30E + 03**	3.51*E* + 03	3.31*E* + 03
	Median	3.30*E* + 03	3.31*E* + 03	**3.26E + 03**	**3.26E + 03**	3.37*E* + 03	**3.26E + 03**
	Mean	3.30*E* + 03	3.31*E* + 03	3.27*E* + 03	**3.26E + 03**	3.37*E* + 03	**3.26E + 03**
	Std	1.69*E* + 01	3.82*E* + 01	1.89*E* + 01	**8.18E + 00**	4.30*E* + 01	1.49*E* + 01
	*P*	1.73*E* − 06(+)	8.35*E* − 08(+)	3.18*E* − 03(+)	9.06*E* − 08(−)	7.39*E* − 11(+)	

*F*_29_(*X*)	Best	4.07*E* + 03	3.90*E* + 03	3.35*E* + 03	3.36*E* + 03	4.99*E* + 03	**3.34E + 03**
	Worst	5.69*E* + 03	5.59*E* + 03	4.01*E* + 03	**3.93E + 03**	6.57*E* + 03	3.99*E* + 03
	Median	4.75*E* + 03	4.75*E* + 03	3.77*E* + 03	**3.68E + 03**	5.78*E* + 03	3.70*E* + 03
	Mean	4.84*E* + 03	4.80*E* + 03	3.74*E* + 03	**3.65E + 03**	5.80*E* + 03	3.69*E* + 03
	Std	3.75*E* + 02	4.58*E* + 02	1.60*E* + 02	1.66*E* + 02	4.30*E* + 02	**1.50E + 02**
	*P*	3.02*E* − 11(+)	3.69*E* − 11(+)	1.76*E* − 01(=)	3.79*E* − 01(=)	3.02*E* − 11(+)	

*F*_30_(*X*)	Best	6.92*E* + 05	6.25*E* + 05	6.18*E* + 05	6.05*E* + 05	2.64*E* + 07	**5.88E + 05**
	Worst	2.24*E* + 06	2.30*E* + 06	**7.72E + 05**	8.91*E* + 05	7.04*E* + 07	7.79*E* + 05
	Median	1.27*E* + 06	1.11*E* + 06	6.94*E* + 05	6.32*E* + 05	3.43*E* + 07	**6.13E + 05**
	Mean	1.31*E* + 06	1.17*E* + 06	6.92*E* + 05	6.44*E* + 05	3.67*E* + 07	**6.31E + 05**
	Std	4.24*E* + 05	3.82*E* + 05	4.34*E* + 04	5.26*E* + 04	4.30*E* + 01	**5.23E + 04**
	*P*	5.49*E* − 11(+)	1.61*E* − 10(+)	5.46*E* − 06(+)	2.42*E* − 02(+)	3.02*E* − 11(+)	
**+/** **=** /−		26/3/0	25/4/0	22/4/3	10/12/7	29/0/0	

**Table 8:** Statistics table of the optimization route by the algorithm.

Map size	Performance index	LSSA	SSA
15 ∗ 15	Shortest	19.7990	25.4558
	Average	21.6846	32.9983
	Worst	25.4558	39.5980

## Data Availability

The data used to support the findings of this study are available from the corresponding author upon request.

## References

[1] Feng Y., Deb S., Wang G. G. (2020). Monarch butterfly optimization: a comprehensive review. *Expert Systems with Applications*.

[2] Li S., Chen H., Wang M., Heidari A. A., Mirjalili S. (2020). Slime mould algorithm: a new method for stochastic optimization. *Future Generation Computer Systems*.

[3] Wang G.-G. (2018). Moth search algorithm: a bio-inspired metaheuristic algorithm for global optimization problems. *Memetic Computing*.

[4] Yang Y., Chen H., Heidari A. A., Gandomi A. H. (2021). Hunger games search: visions, conception, implementation, deep analysis, perspectives, and towards performance shifts. *Expert Systems with Applications*.

[5] Salgotra R., Singh U. (2019). The naked mole-rat algorithm. *Neural Computing and Applications*.

[6] Heidari A. A., Mirjalili S., Faris H., Aljarah I., Mafarja M., Chen H. (2019). Harris hawks optimization: algorithm and applications. *Future Generation Computer Systems*.

[7] Xue J., Shen B. (2020). A novel swarm intelligence optimization approach: sparrow search algorithm. *Systems Science & Control Engineering*.

[8] Mirjalili S., Mirjalili S. M., Lewis A. (2014). Grey wolf optimizer. *Advances in Engineering Software*.

[9] Kennedy J., Eberhart R. C. A discrete binary version of the particle swarm algorithm.

[10] Houck C. R., Joines J., Kay. M. G. (1995). A genetic algorithm for function optimization: a Matlab implementation. *Ncsu-ie Tr*.

[11] Lu X., Mu X., Zhang J., Wang Z. (2020). Chaos sparrow search optimization algorithm. *Journal of Beijing University of Aeronautics and Astronautics*.

[12] Lu X., Mu X., Zhang J. (2021). Multi-threshold image segmentation based on improved sparrow search algorithm. *Systems Engineering and Electronics*.

[13] Mao Q., Zhang Q. (2020). Improved sparrow algorithm combining Cauchy mutation and opposition-based learning. *Journal of Computer Science and Exploration*.

[14] Liu G., Shu C., Liang Z., Peng B., Cheng L. (2021). A modified sparrow search algorithm with application in 3D route planning for UAV. *Sensors*.

[15] Wang P., Zhang Y., Yang H. (2021). Research on economic optimization of microgrid cluster based on chaos sparrow search algorithm. *Computational Intelligence and Neuroscience*.

[16] Zhang C., Ding S. (2021). A stochastic configuration network based on chaotic sparrow search algorithm. *Knowledge-Based Systems*.

[17] Wang T., Yang L. (2018). Beetle swarm optimization algorithm: theory and application. https://arxiv.org/abs/1808.00206.

[18] Peng H., Zeng Z., Deng C., Wu Z. (2021). Multi-strategy serial cuckoo search algorithm for global optimization. *Knowledge-Based Systems*.

[19] Salgotra R., Singh U., Saha S. Improving cuckoo search: incorporating changes for CEC 2017 and CEC 2020 benchmark problems.

[20] Peng H., Zhu W., Deng C., Wu Z. (2021). Enhancing firefly algorithm with courtship learning. *Information Sciences*.

[21] Li W., Wang G. G., Gandomi A. H. (2021). A survey of learning-based intelligent optimization algorithms. *Archives of Computational Methods in Engineering*.

[22] Li W., Wang G.-G., Alavi A. H. (2020). Learning-based elephant herding optimization algorithm for solving numerical optimization problems. *Knowledge-Based Systems*.

[23] Li W., Wang G. G. (2021). Elephant herding optimization using dynamic topology and biogeography-based optimization based on learning for numerical optimization. *Engineering with Computers*.

[24] Tizhoosh H. R. (2005). Opposition-based learning: a new scheme for machine intelligence. *International Conference on Computational Intelligence for Modelling, Control and Automation and International Conference on Intelligent Agents, Web Technologies and Internet Commerce (CIMCA-IAWTIC’06)*.

[25] He J., Peng Z., Cui D., Li Q. (2019). A teaching and learning optimization algorithm based on multi-inverse learning. *Engineering Science and Technology*.

[26] Rahnamayan S., Tizhoosh H. R., Salama M. M. A. (2008). Opposition-based differential evolution. *IEEE Transactions on Evolutionary Computation*.

[27] Wen L., Wu T., Tang M. (2020). Gray wolf optimization algorithm based on lens imaging learning strategy. *Acta Automatica Sinica*.

[28] Mirjalili S. (2016). SCA: a sine cosine algorithm for solving optimization problems. *Knowledge-based Systems*.

[29] Sindhu R., Ngadiran R., Yacob Y. M., Zahri N. A. H., Hariharan M. (2017). Sine-cosine algorithm for feature selection with elitism strategy and new updating mechanism. *Neural Computing and Applications*.

[30] Ouyang C., Zhu D. (2021). Multi-strategy improved sparrow search algorithm based on K-means. *Electro-Optics and Control*.

[31] Fengtao W., Zhang Y., Li J., Shi Y. (2021). Improved sine and cosine algorithm based on dynamic classification strategy. *System Engineering and Electronic Technology*.

[32] Yu Li, Zhao Y., Liu J. (2021). A levy flight sine cosine algorithm for global optimization problems. *International Journal of Distributed Systems and Technologies (IJDST)*.

[33] Luo J., Liu Z., Zhang P., Liu X., Zheng L. (2020). The application of improved bird swarm algorithm based on nonlinear factors in dynamic energy consumption management. *Journal of Electronics & Information Technology*.

[34] Awad N. H., Ali M. Z., Liang J. J. (2016). Problem definitions and evaluation criteria for the CEC 2017 special session and competition on single objective real-parameter numerical optimization.

